RETRACTED

# Associations of vitamin D receptor polymorphisms with risk of Alzheimer’s disease, Parkinson’s disease, and mild cognitive impairment: a systematic review and meta-analysis

**DOI:** 10.3389/fnagi.2024.1377058

**Published:** 2024-04-12

**Authors:** Yanjun Du, Peizhen Geng, Qunqun Chen, Laixi Han, Lu Liu, Maoquan Yang, Mingzhu Tan, Jun Meng, Xiaojuan Sun, Lidan Feng

**Affiliations:** ^1^Department of Encephalopathy, Weifang Hospital of Traditional Chinese Medicine, Weifang, Shandong, China; ^2^School of Clinical Medicine, Shandong Second Medical University, Weifang, Shandong, China; ^3^Department of Rehabilitation, Weifang Brain Hospital, Weifang, Shandong, China; ^4^Department of Occupational Diseases, Weifang People’s Hospital, Weifang, Shandong, China; ^5^Department of Rehabilitation, Weifang People’s Hospital, Weifang, Shandong, China

**Keywords:** Alzheimer’s disease, Parkinson’s disease, mild cognitive impairment, VDR, gene polymorphism, susceptibility, meta-analysis

## Abstract

Vitamin D is a lipid soluble steroid hormone, which plays a critical role in the calcium homeostasis, neuronal development, cellular differentiation, and growth by binding to vitamin D receptor (VDR). Associations between VDR gene polymorphism and Alzheimer’s disease (AD), Parkinson’s disease (PD), and mild cognitive impairment (MCI) risk has been investigated extensively, but the results remain ambiguous. The aim of this study was to comprehensively assess the correlations between four VDR polymorphisms (*Fok*I, *Bsm*I, *Taq*I, and *Apa*I) and susceptibility to AD, PD, and MCI. Crude odds ratios (ORs) and 95% confidence intervals (CIs) were calculated to determine the relationship of interest. Pooled analyses suggested that the *Apa*I polymorphism decreased the overall AD risk, and the *Taq*I increased the overall PD susceptibility. In addition, the *Bsm*I and *Apa*I polymorphisms were significantly correlated with the overall MCI risk. Stratified analysis by ethnicity further showed that the *Taq*I and *Apa*I genotypes reduced the AD predisposition among Caucasians, while the *Taq*I polymorphism enhanced the PD risk among Asians. Intriguingly, carriers with the BB genotype significantly decreased the MCI risk in Asian descents, and the *Apa*I variant elevated the predisposition to MCI in Caucasians and Asians. Further studies are need to identify the role of VDR polymorphisms in AD, PD, and MCI susceptibility.

## 1 Introduction

Alzheimer’s disease (AD), a chronic neurodegenerative disorder, is the most common cause of irreversible disability and dementia in the elderly, presenting with progressive memory decline and cognitive impairment (Hodson, 2018; Zhang et al., 2023). The prevalence of dementia is estimated to double every 20 years, and the global number could increase to 131.5 million by 2050, causing a huge economic burden and affecting the quality of life (Tolosa et al., 2021). Parkinson’s disease (PD) is the second most common neurodegenerative disease after AD, which is characterized by resting tremor, rigidity, bradykinesia, postural instability, and freezing of gait, affecting nearly 1.7% of the population older than age 65 years (Samii et al., 2004; de Lau and Breteler, 2006). Mechanistically, the pathology of AD is characterized by abnormal amyloid-β (Aβ) deposition, hyperphosphorylated Tau formation of neurofibrillary tangles, and neuroinflammation (Scheff et al., 2006; Nelson et al., 2012; Hamilton et al., 2022). The hallmarks of PD are degeneration of dopaminergic neurons in the substantia nigra pars compact and aggregation of the misfolded α-synuclein in the intracellular inclusions known as Lewy bodies (Braak et al., 2003; Surmeier et al., 2017). Mild cognitive impairment (MCI) is a transitional state between normal aging and dementia. Studies have shown that MCI at a high conversion rate was prone to develop into dementia, providing a novel strategy for the prevention, prognosis and treatment of AD and PD (Gauthier et al., 2006; Hansson et al., 2006; Petersen, 2018). It is widely believed that environmental exposures and genetic factors influenced the susceptibility to environmental factors, including smoking, alcohol, obesity, diabetes, drug abuse, poor diet, and physical inactivity. Therefor, gene-environment interactions may be implicated in the pathogenesis of neurodegenerative diseases (Panza et al., 2008; Durazzo et al., 2014; Polidori, 2014; Silva et al., 2019; Periñán et al., 2022).

RETRACTED

Accumulative evidence has demonstrated that serum vitamin D deficiency is inversely associated with the risk of several neurodegenerative diseases, such as MCI, AD, and PD (Suzuki et al., 2012; Wang et al., 2012, 2015; Koduah et al., 2017). It has been reported that vitamin D supplements could effectively prevent deterioration of diseases and improve cognitive function (Peterson et al., 2013; Suzuki et al., 2013). Vitamin D belongs to a group of lipid soluble steroid hormone (Norman, 1998). It is primarily synthesized by the skin via exposure to sunlight, and a small portion is absorbed from dietary sources. The 25-hydroxy vitamin D3 stored in the kidneys is metabolized by 1-α-hydroxylase and converts into biologically active 1,25-dihydroxyvitamin D3. The active metabolite regulates transcription of targeted vitamin D-responsive genes by interacting with nuclear vitamin D receptor (VDR), and then exerts its biological function, including cell cycle activity, calcium homeostasis, stress response, immunoregulation, neuronal development, cellular differentiation, and growth (Haussler et al., 1998; Bouillon et al., 2008; Cesari et al., 2011). Being highly expressed in the hypothalamus and substantia nigra, VDR is a member of nuclear steroid hormone receptor superfamily (Eyles et al., 2005, 2013; Kesby et al., 2011), and VDR knockout mice had muscular and motor impairments (Burne et al., 2005). As a consequence, VDR gene polymorphisms may influence the VDR expression, structure, and function.

RETRACTED

The VDR gene is located on chromosome 12 (12q13.11), consisting of two promoter regions, eight exons and seven introns that span more than 100 kb in length (Albert et al., 2009; Bollen et al., 2022). Up to now, genome-wide association studies (GWAs) have identified several hazard VDR gene single nucleotide polymorphisms (SNPs) (Beecham et al., 2009). Among these VDR SNPs, the *Fok*I (rs2228570) at exon 2 on the 5′ coding region is a functional polymorphism where the alteration of T to C produces a shorter protein with higher transcription capacity, and has no linkage with any of other VDR gene polymorphisms (Gross et al., 1998). The *Bsm*I (rs1544410), *Apa*I (rs7975232), and *Taq*I (rs731236) are situated near the 3′ untranslated region (UTR) of VDR gene (Morrison et al., 1994). These SNPs could impact on the stability and translation efficiency of VDR mRNA, but not structurally change its amino acid sequence (Uitterlinden et al., 2004). Moreover, they have strong linkage disequilibrium with variants in the 3′UTR, which favors the modulation of VDR gene expression (Ingles et al., 1997; Zmuda et al., 2000).

Numerous studies have investigated the associations of VDR gene SNPs wit AD, MCI, and PD risk, but the results remain inconsistent and controversial. Lee et al. (2014) proved that VDR *Bsm*I polymorphism was correlated with PD risk among Asians, as well as the *Fok*I. Another study found that the *Bsm*I significantly increased the risk of MCI, and the *Taq*I was positively correlated with the AD risk, while the *Apa*I reduced the susceptibility to MCI (Liu et al., 2021). Han et al. (2012) reported that the *Fok*I CC + CT genotype was remarkably associated with sporadic PD risk in the Chinese population. Recent study have shown that the *Fok*I SNP, but not *Bsm*I, *Apa*I, or *Taq*I, was significantly correlative with PD susceptibility (Török et al., 2013; Zhang et al., 2014). Inversely, Gezen-Ak et al. (2012) demonstrated that the Aa genotype significantly elevated the risk of developing AD 2.3 times compared with the *Apa*I AA genotype. The *Taq*I G-allele has been reported to be correlative with greater cognitive decline (Kuningas et al., 2009). Due to the small sample size and limited number of gene loci included in the study, we performed this meta-analysis to accurately evaluate the correlation between VDR SNPs (*Fok*I, *Bsm*I, *Apa*I, and *Taq*I) and susceptibility to AD, MCI, and PD.

RETRACTED

## 2 Materials and methods

### 2.1 Literature search strategy

This meta-analysis was performed according to the Preferred Reporting Items for Systematic Reviews and Meta-Analyses (PRISMA) guidelines (Moher et al., 2009). Eligible studies were extracted from the PubMed, EMBASE, Web of Science, and Cochrane Library databases up to date to 22 September 2023. Our search strategy included the following terms (Alzheimer’s disease or AD or Parkinson’s disease or PD or mild cognitive impairment or MCI) and (vitamin D receptor or VDR) and (polymorphism or SNP or genotype or mutation or variant). At the same time, the selected potential articles were manually screened out in the cited references.

### 2.2 Selection and exclusion criteria

Inclusion criteria are as follows: (1) case-control studies investigated the association between VDR polymorphisms and susceptibility to AD, PD, and MCI; (2) the patients were diagnosed clinically by the neurologist in accordance of DSMIV criteria, the United Kingdom Parkinson’s Disease Brain Bank criteria and the Hoehn and Yahr Scale; and (3) the sufficient information on genotypic distribution of VDR gene. The exclusion criteria were as follows: (1) non-case-control study; (2) animal studies; (3) review, abstract, case reports, meta-analysis, comments, and editorials; (4) lack of detailed genotyping data; and (5) other gene type and additional VDR genotype.

### 2.3 Data extraction

Two experienced authors (YD and PG) independently conducted literature screening, data extraction, literature quality evaluation, and any disagreements could be resolved through discussion or a third analyst (XS). The detailed information extracted from all the selected studies included: first author’s surname, publication year, country, type of disease, ethnicity, source of controls, genotyping methods, sample size, and *P*-value of HWE.

The Newcastle-Ottawa Scale (NOS) was used to evaluate the process in terms of queue selection, comparability of queues, and evaluation of results (Stang, 2010). A study with a score of at least six was considered as a high-quality literature. Higher NOS scores showed higher literature quality.

### 2.4 Statistical analysis

All data analysis was conducted using Stata16.0 software (Stata Corp LP, TX, USA). Odds ratio (OR) and 95% confidence intervals (CIs) were used to assess the correlations of VDR gene polymorphisms with AD, PD, and MCI risk. After that, the heterogeneity test was carried out. The *P* ≥ 0.05 or *I*^2^ < 50% suggested no distinct heterogeneity, and the fixed-effect pattern was applied to integrate the results. Otherwise, the random-effect model was used. Results were considered significant statistically when the *P*-value less than 0.05. Subsequently, we carried out the subgroup analysis in order to determine the source of heterogeneity. In addition, sensitivity analysis was performed by removing one study sequentially to evaluate the influence of each individual study on overall results under all genetic models. Among these studies, the publication bias was verified by using the Begg’s rank correlation test and Egger’s linear regression test. If *P* < 0.05 indicates obvious publication bias.

RETRACTED

### 2.5 False-positive report probability analysis

The probability of meaningful associations between VDR SNPs and the risk of AD, PD, and MCI can be determined by conducting the false-positive report probability (FPRP) analysis (Wacholder et al., 2004). In order to explore the relationships observed in the meta-analysis, we adopted prior probabilities of 0.25, 0.1, 0.01, 0.001, and 0.0001 and computed the FPRP values as described previously. The relevance that reached the FPRP threshold of <0.2 was considered significant.

## 3 Results

### 3.1 Literature search and screening

The flow diagram (Figure 1) showed detailed literature search steps. The systematic search yielded 1,369 potential articles retrieved from the initial databases of PubMed (*n* = 1004), Embase (*n* = 98), Web of Science (*n* = 245), Cochrane Library (*n* = 21), and one additional record was retrieved through other sources (Mohammadzadeh and Pazhouhesh, 2016). After exclusion of 168 duplicate references, 1,201 articles were considered for the meta-analysis. Of the remaining 1,201 articles, we removed 914 articles after screening the title and abstract. Among these, 511 articles were reviews, comments, letters, meta-analysis, case report, editorials, cross-sectional studies, conference abstracts, and conference papers, while 403 articles were implicated in animal or *in vitro* studies. At this stage, 287 research literatures were reviewed again. After carefully reviewing the full texts, we performed a secondary screening and eliminated 257 articles due to other disease (*n* = 231), insufficient information (*n* = 3), other genes and VDR gene polymorphisms (*n* = 23). A total of 30 studies covering 81 studies were retained for this meta-analysis (Luedecking-Zimmer et al., 2003; Kim et al., 2005; Gezen-Ak et al., 2007, 2012, 2017; Lehmann et al., 2011; Han et al., 2012; Khorram Khorshid et al., 2013; Liu et al., 2013; Lv et al., 2013; Török et al., 2013; Petersen et al., 2014; Gatto et al., 2015; Łaczmański et al., 2015; Zhou et al., 2015; Kang et al., 2016; Mohammadzadeh and Pazhouhesh, 2016; Mun et al., 2016; Meamar et al., 2017; Tanaka et al., 2017; Oliveira et al., 2018; Hu et al., 2020; Agliardi et al., 2021; Arévalo et al., 2021; Agúndez et al., 2022; Dimitrakis et al., 2022a,b; Kamyshna et al., 2022; Redenšek et al., 2022; Zhang et al., 2022).

RETRACTED

**FIGURE 1:** Flow diagram of the eligible study selection process.

### 3.2 Characteristics of included studies

The main characteristics of all included studies are summarized in Table 1. Seventeen studies were conducted in the Caucasian population, and 13 studies in the Asian population. The control group of 11 studies were population-based (PB), and 19 studies were hospital-based (HB). And then, these studies were assessed by NOS and met the high-quality standards (Supplementary Table 1). Additionally, PCR method was used to measure in 10 studies, PCR-RFLP method in 11 studies, TaqMan method in 6 studies, Snapshot method in 2 studies, and other methods in 2 studies, respectively. As for AD risk, 6 studies of VDR *Fok*I polymorphism, 5 studies of *Bsm*I polymorphism, 7 studies of *Taq*I polymorphism, and 5 studies of *Apa*I polymorphism were analyzed. For the risk of PD, 12 studies on VDR *Fok*I polymorphism, 11 studies on VDR *Bsm*I polymorphism, 12 studies on *Taq*I polymorphism, and 10 studies on VDR *Apa*I polymorphism were enrolled to investigate the association. With regard to the risk of MCI, three studies focused on the *Fok*I SNP, three studies on the *Bsm*I SNP, three studies on the *Taq*I SNP, and four studies on the *Apa*I SNP in this meta-analysis (Table 2).

**TABLE 1:** Summary characteristics of the included studies in our meta-analysis.

References	Country	Ethnicity	Disease	Sample size case/control	Genotyping methods	Source of control	NOS	VDR SNPs
Luedecking-Zimmer et al., 2003	USA	Caucasian	AD	564/492	PCR	HB	6	*Fok*I
Kim et al., 2005	Korea	Asian	PD	85/231	PCR-RFLP	HB	6	*Bsm*I
Gezen-Ak et al., 2007	Turkey	Caucasian	AD	104/109	PCR	HB	6	*Taq*I, *Apa*I
Lehmann et al., 2011	UK	Caucasian	AD	255/260	PCR	PB	7	*Taq*I, *Apa*I
Han et al., 2012	China	Asian	PD	260/282	PCR-RFLP	HB	6	*Fok*I, *Bsm*I
Gezen-Ak et al., 2012	UK	Caucasian	AD	108/112	PCR	HB	6	*Fok*I, *Bsm*I, *Tru*9I
Török et al., 2013	Hungary	Caucasian	PD	100/109	PCR	HB	6	*Fok*I, *Bsm*I, *Taq*I, *Apa*I
Liu et al., 2013	China	Asian	PD	285/285	PCR-RFLP	HB	7	*Taq*I, *Apa*I
Khorram Khorshid et al., 2013	Iran	Asian	AD	145/162	PCR-RFLP	PB	8	*Taq*I, *Apa*I
Lv et al., 2013	China	Asian	PD	498/483	PCR	PB	7	*Taq*I
Petersen et al., 2014	Denmark	Caucasian	PD	121/235	PCR	HB	8	*Bsm*I, *Taq*I, *Apa*I
Zhou et al., 2015	China	Asian	MCI	124/124	SNaPshot	PB	7	*Bsm*I, *Apa*I
Łaczmański et al., 2015	Poland	Caucasian	AD	108/77	SNaPshot	HB	6	*Fok*I, *Bsm*I, *Taq*I
Gatto et al., 2015	USA	Caucasian	PD	283/419	TaqMan	PB	9	*Fok*I, *Bsm*I, *Taq*I, *Apa*I, Cdx-2
Mohammadzadeh and Pazhouhesh, 2016	Iran	Asian	PD	150/160	PCR-RFLP	HB	6	*Fok*I, *Apa*I,
Kang et al., 2016	Korea	Asian	PD	137/163	PCR	PB	7	*Fok*I, *Bsm*I, *Taq*I
Mun et al., 2016	Korea	Asian	AD	144/329	PCR	PB	7	*Fok*I, *Bsm*I, *Taq*I, *Apa*I
Meamar et al., 2017	Iran	Asian	PD	59/53	PCR-RFLP	HB	6	*Fok*I, *Bsm*I, *Taq*I, *Apa*I,
Tanaka et al., 2017	Japan	Asian	PD	298/250	TaqMan	HB	6	*Fok*I, *Bsm*I, *Taq*I, *Apa*I
Gezen-Ak et al., 2017	Turkey	Caucasian	PD	382/242	PCR-RFLP	HB	7	*Fok*I, *Bsm*I, *Taq*I, *Apa*I, *Tru*9I
Oliveira et al., 2018	Brazil	Caucasian	AD/MCI	32/24	PCR-RFLP	HB	7	*Fok*I, *Bsm*I, *Taq*I, *Apa*I
Hu et al., 2020	China	Asian	PD	470/470	PCR	PB	8	*Fok*I
Arévalo et al., 2021	Chile	Caucasian	MCI	66/128	TaqMan	HB	7	*Taq*I, *Apa*I
Agliardi et al., 2021	Italy	Caucasian	PD	406/800	TaqMan	PB	9	*Fok*I, *Bsm*I, *Taq*I, *Apa*I
Agúndez et al., 2022	Spain	Caucasian	PD	272/272	TaqMan	PB	7	*Fok*I, *Taq*I, *Apa*I
Dimitrakis et al., 2022a	Greece	Caucasian	AD	90/103	PCR-RFLP	HB	6	*Fok*I, *Bsm*I, *Taq*I
Dimitrakis et al., 2022b	Greece	Caucasian	AD	90/103	PCR-RFLP	HB	6	*Taq*I
Zhang et al., 2022	China	Asian	MCI	171/261	PCR-RFLP	PB	9	*Fok*I, *Bsm*I, *Taq*I, *Apa*I
Kamyshna et al., 2022	Ukraine	Caucasian	MCI	53/125	TaqMan	HB	7	*Fok*I
Redenšek et al., 2022	Slovenia	Caucasian	PD	231/161	KASPar	HB	7	*Fok*I, *Bsm*I, *Taq*I, Cdx-2

PB, population-based; HB, hospital-based; PCR-RFLP, polymerase chain reaction-restriction fragment length polymorphism; AD, Alzheimer’s disease; MCI, mild cognitive impairment; PD, Parkinson’s disease; NOS, Newcastle-Ottawa Scale; SNP, single nucleotide polymorphism.

RETRACTED

**TABLE 2:** Genotype frequencies of vitamin D receptor SNPs in AD, MCI, and PD patients and matched controls.

References	Country	Case			Control			HWE
		**AA**	**Aa**	**aa**	**AA**	**Aa**	**aa**	***P*-value**
**6 studies for VDR FokI polymorphism in AD**								
Luedecking-Zimmer et al., 2003	USA	233	225	78	198	229	65	0.9243
Gezen-Ak et al., 2012	UK	52	46	10	51	51	10	0.5847
Łaczmański et al., 2015	Poland	36	53	19	27	36	14	0.7421
Mun et al., 2016	Korea	43	77	24	129	148	52	0.3823
Oliveira et al., 2018	Brazil	15	14	3	12	11	1	0.4319
Dimitrakis et al., 2022a	Greece	55	38	10	34	39	5	0.1566
**5 studies for VDR BsmI polymorphism in AD**								
Gezen-Ak et al., 2012	UK	39	38	30	48	32	34	0.0000
Łaczmański et al., 2015	Poland	35	61	12	23	44	10	0.1217
Mun et al., 2016	Korea	125	19	0	294	34	1	0.9871
Oliveira et al., 2018	Brazil	12	11	9	10	12	2	0.5403
Dimitrakis et al., 2022a	Greece	33	51	19	30	26	22	0.0040
**7 studies for VDR TaqI polymorphism in AD**								
Gezen-Ak et al., 2007	Turkey	38	50	16	53	39	17	0.0399
Lehmann et al., 2011	UK	101	117	42	68	136	51	0.2540
Łaczmański et al., 2015	Poland	42	55	11	31	38	8	0.0058
Mun et al., 2016	Korea	125	19	0	296	32	1	0.8912
Oliveira et al., 2018	Brazil	10	11	11	7	6	2	0.6985
Dimitrakis et al., 2022a	Greece	38	32	8	35	49	19	0.7996
Dimitrakis et al., 2022b	Greece	44	37	9	35	49	19	0.7996
**5 studies for VDR ApaI polymorphism in AD**								
Gezen-Ak et al., 2007	Turkey	54	74	49	52	109	43	0.3125
Lehmann et al., 2011	UK	250	195	55	284	178	38	0.1754
Khorram Khorshid et al., 2013	Iran	583	462	102	666	462	75	0.8848
Mun et al., 2016	Korea	552	418	79	729	565	103	0.6510
Oliveira et al., 2018	Brazil	237	220	39	99	80	27	0.0982
**12 studies for VDR FokI polymorphism in PD**								
Han et al., 2012	China	114	124	22	109	126	47	0.3057
Török et al., 2013	Hungary	42	48	10	35	49	25	0.3301
Gatto et al., 2015	USA	109	126	48	153	203	66	0.9216
Mohammadzadeh and Pazhouhesh, 2016	Iran	123	27	0	134	26	0	0.2633
Kang et al., 2016	Korea	46	63	28	48	79	36	0.7458
Meamar et al., 2017	Iran	6	22	31	2	11	40	0.2885
Tanaka et al., 2017	Japan	108	98	23	141	169	47	0.7691
Gezen-Ak et al., 2017	Turkey	181	164	37	105	107	25	0.7691
Hu et al., 2020	China	131	220	119	149	243	78	0.2071
Agliardi et al., 2021	Italy	136	196	74	362	343	95	0.3221
Redenšek et al., 2022	Slovenia	88	102	41	84	17	58	0.0000
Agúndez et al., 2022	Spain	117	128	27	110	124	38	0.7473
**11 studies for VDR BsmI polymorphism in PD**								
Kim et al., 2005	Korea	72	11	2	168	60	3	0.3570
Han et al., 2012	China	4	34	222	2	36	244	0.5992
Török et al., 2013	Hungary	27	49	24	27	57	25	0.6294
Petersen et al., 2014	Denmark	48	53	20	84	117	34	0.5102
Gatto et al., 2015	USA	79	161	36	151	215	50	0.0448
Kang et al., 2016	Korea	123	13	1	145	17	1	0.5242
Meamar et al., 2017	Iran	8	27	24	8	28	17	0.5279
Tanaka et al., 2017	Japan	178	45	6	291	60	6	0.1666
Gezen-Ak et al., 2017	Turkey	136	134	110	94	78	67	0.0000
Agliardi et al., 2021	Italy	131	167	108	276	307	217	0.0000
Redenšek et al., 2022	Slovenia	78	119	34	58	72	30	0.3658
**12 studies for VDR TaqI polymorphism in PD**								
Lv et al., 2013	China	446	52	0	437	46	0	0.2718
Török et al., 2013	Hungary	35	48	17	47	46	16	0.3938
Liu et al., 2013	China	20	135	130	24	112	149	0.6506
Petersen et al., 2014	Denmark	47	54	20	81	119	34	0.3599
Gatto et al., 2015	USA	77	162	43	153	213	55	0.1518
Kang et al., 2016	Korea	22	78	37	30	73	48	0.8137
Meamar et al., 2017	Iran	6	25	28	4	26	23	0.3597
Tanaka et al., 2017	Japan	178	47	4	284	67	6	0.3808
Gezen-Ak et al., 2017	Turkey	154	182	45	109	98	33	0.1527
Agliardi et al., 2021	Italy	134	208	64	288	385	127	0.9295
Redenšek et al., 2022	Slovenia	84	113	34	72	29	60	0.0000
Agúndez et al., 2022	Spain	110	125	37	86	139	47	0.4730
**10 studies for VDR ApaI polymorphism in PD**								
Török et al., 2013	Hungary	15	43	42	21	46	42	0.1975
Liu et al., 2013	China	252	33	0	255	30	0	0.3483
Petersen et al., 2014	Denmark	25	62	34	56	120	58	0.6940
Gatto et al., 2015	USA	78	158	46	105	210	104	0.9609
Mohammadzadeh and Pazhouhesh, 2016	Iran	36	84	30	128	27	5	0.0270
Meamar et al., 2017	Iran	14	32	13	2	34	17	0.0041
Tanaka et al., 2017	Japan	109	102	18	169	156	32	0.6383
Gezen-Ak et al., 2017	Turkey	57	194	130	25	115	101	0.3537
Agliardi et al., 2021	Italy	105	183	118	162	394	244	0.8978
Agúndez et al., 2022	Spain	56	146	69	51	137	84	0.7118
**3 studies for VDR FokI polymorphism in MCI**								
Oliveira et al., 2018	Brazil	6	8	1	12	11	1	0.4319
Zhang et al., 2022	China	72	142	47	49	83	39	0.7348
Kamyshna et al., 2022	Ukraine	11	23	19	26	50	49	0.0547
**3 studies for VDR BsmI polymorphism in MCI**								
Zhou et al., 2015	China	8	47	69	2	33	89	0.5908
Oliveira et al., 2018	Brazil	6	7	2	10	12	2	0.5403
Zhang et al., 2022	China	221	39	1	123	47	1	0.1178
**3 studies for VDR TaqI polymorphism in MCI**								
Oliveira et al., 2018	Brazil	7	6	2	7	6	2	0.6985
Arévalo et al., 2021	Chile	53	53	22	32	31	3	0.1832
Zhang et al., 2022	China	241	20	0	154	16	1	0.4195
**4 studies for VDR ApaI polymorphism in MCI**								
Zhou et al., 2015	China	32	63	29	49	58	17	0.9802
Oliveira et al., 2018	Brazil	1	8	6	2	13	9	0.3672
Arévalo et al., 2021	Chile	34	48	46	23	32	11	0.9815
Zhang et al., 2022	China	137	104	20	95	63	13	0.7263

AD, Alzheimer’s disease; MCI, mild cognitive impairment; PD, Parkinson’s disease; AA, homozygote; Aa, common heterozygote; aa, rare homozygote; HWE, Hardy–Weinberg equilibrium; SNP, single nucleotide polymorphism. *P < 0.05.

RETRACTED

### 3.3 Associations of VDR gene polymorphisms with AD risk

Six articles with 1,031 cases and 1,112 controls explored correlation between VDR *Fok*I polymorphism and the AD risk, five studies with 494 cases and 622 controls detected correlation between VDR *Bsm*I polymorphism and the AD risk, seven studies with 816 cases and 991 controls examined relationship between VDR *Taq*I polymorphism and the AD risk, and five literatures involving 685 cases and 879 controls investigated association between VDR *Apa*I polymorphism and the AD risk. As for VDR *Fok*I (f vs. F: OR = 1.01, 95% CI = 0.89–1.15, *P* = 0.850; ff vs. FF: OR = 1.11, 95% CI = 0.84–1.46, *P* = 0.456; Ff vs. FF: OR = 0.94, 95% CI = 0.78–1.13, *P* = 0.525; ff/Ff vs. FF: OR = 0.97, 95% CI = 0.82–1.16, *P* = 0.753; ff vs. Ff/FF: OR = 1.11, 95% CI = 0.86–1.44, *P* = 0.407, Supplementary Figure 1) and *Bsm*I polymorphisms (B vs. b: OR = 1.05, 95% CI = 0.85–1.29, *P* = 0.655; BB vs. bb: OR = 1.01, 95% CI = 0.66–1.54, *P* = 0.960; Bb vs. bb: OR = 1.27, 95% CI = 0.94–1.73, *P* = 0.125; BB/Bb vs. bb: OR = 1.19, 95% CI = 0.89–1.58, *P* = 0.243; BB vs. Bb/bb: OR = 0.88, 95% CI = 0.60–1.28, *P* = 0.491, Supplementary Figure 2), we did not find any prominent associations in overall and subgroup analyses. The overall pooled results manifested that VDR *Taq*I polymorphism was dramatically relevant to AD risk under homozygous model (tt vs. TT: OR = 0.67, 95% CI = 0.49–0.93, *P* = 0.017, Supplementary Figure 3), and the *Apa*I polymorphism was significantly correlated with AD risk under allelic, homozygous, and recessive models (A vs. a: OR = 0.85, 95% CI = 0.73–0.99, *P* = 0.033; AA vs. aa: OR = 0.68, 95% CI = 0.47–0.96, *P* = 0.030; AA vs. Aa/aa: OR = 0.72, 95% CI = 0.56–0.92, *P* = 0.009, Figure 2 and Table 3).

**FIGURE 2:** Forest plots for the association between VDR *Apa*I polymorphism and AD risk in five models. **(A)** Allele model; **(B)** homozygote model; **(C)** heterozygote model; **(D)** dominant model; **(E)** recessive model.

**TABLE 3:** Meta-analysis results for the relationship of VDR gene SNPs with AD, MCI, and PD risk.

SNP	Model	OR (95% CI)	*P*	*I*^2^ (%)	*P*_(*H*)_	Effect model
**AD**						
*Fok*I	Allelic (f vs. F)	1.01 (0.89, 1.15)	0.850	0.0	0.685	FEM
	Homozygous (ff vs. FF)	1.11 (0.84, 1.46)	0.456	0.0	0.939	FEM
	Heterozygous (Ff vs. FF)	0.94 (0.78, 1.13)	0.525	38.5	0.149	FEM
	Dominant (ff/Ff vs. FF)	0.97 (0.82, 1.16)	0.753	25.5	0.243	FEM
	Recessive (ff vs. FF/Ff)	1.11 (0.86, 1.44)	0.407	0.0	0.965	FEM
*Bsm*I	Allelic (B vs. b)	1.05 (0.85, 1.29)	0.655	0.0	0.674	FEM
	Homozygous (BB vs. bb)	1.01 (0.66, 1.54)	0.960	0.0	0.580	FEM
	Heterozygous (Bb vs. bb)	1.27 (0.94, 1.73)	0.125	0.0	0.581	FEM
	Dominant (BB/Bb vs. bb)	1.19 (0.89, 1.58)	0.243	0.0	0.903	FEM
	Recessive (BB vs. bb/Bb)	0.88 (0.60, 1.28)	0.491	20.6	0.283	FEM
*Taq*I	Allelic (t vs. T)	0.91 (0.69, 1.21)	0.534	65.9	0.007	REM
	Homozygous (tt vs. TT)	0.67 (0.49, 0.93)	0.017*	42.2	0.109	FEM
	Heterozygous (Tt vs. TT)	0.91 (0.63, 1.34)	0.639	61.5	0.016	REM
	Dominant (tt/Tt vs. TT)	0.90 (0.60, 1.33)	0.584	68.1	0.008	REM
	Recessive (tt vs. TT/Tt)	0.78 (0.58, 1.05)	0.104	0.0	0.459	FME
*Apa*I	Allelic (A vs. a)	0.85 (0.73, 0.99)	0.033*	6.2	0.371	FME
	Homozygous (AA vs. aa)	0.68 (0.47, 0.96)	0.030*	0.0	0.518	FME
	Heterozygous (Aa vs. aa)	0.88 (0.58, 1.34)	0.809	36.8	0.176	FEM
	Dominant (AA/Aa vs. aa)	0.90 (0.70, 1.15)	0.390	26.5	0.245	FEM
	Recessive (AA vs. aa/Aa)	0.72 (0.56, 0.92)	0.009*	27.5	0.238	FME
**PD**						
*Fok*I	Allelic (f vs. F)	0.92 (0.77, 1.08)	0.304	78.2	0.000	REM
	Homozygous (ff vs. FF)	0.81 (0.56, 1.16)	0.248	79.2	0.000	REM
	Heterozygous (Ff vs. FF)	1.09 (0.85, 1.39)	0.507	76.4	0.000	REM
	Dominant (ff/Ff vs. FF)	0.99 (0.82, 1.21)	0.955	68.7	0.000	REM
	Recessive (ff vs. FF/Ff)	0.76 (0.53, 1.09)	0.136	83.2	0.000	REM
*Bsm*I	Allelic (B vs. b)	1.05 (0.96, 1.14)	0.326	0.0	0.601	FEM
	Homozygous (BB vs. bb)	1.09 (0.91, 1.31)	0.367	0.0	0.964	FEM
	Heterozygous (Bb vs. bb)	1.09 (0.95, 1.25)	0.240	26.2	0.194	FEM
	Dominant (BB/Bb vs. bb)	1.09 (0.95, 1.24)	0.219	16.2	0.290	FEM
	Recessive (BB vs. bb/Bb)	1.02 (0.87, 1.19)	0.818	0.0	0.960	FEM
*Taq*I	Allelic (t vs. T)	1.00 (0.93, 1.09)	0.951	32.2	0.133	FEM
	Homozygous (tt vs. TT)	0.96 (0.80, 1.14)	0.607	32.0	0.143	FEM
	Heterozygous (Tt vs. TT)	1.24 (0.99, 1.54)	0.057	63.6	0.001	REM
	Dominant (tt/Tt vs. TT)	1.13 (1.01, 1.27)	0.033*	29.1	0.160	FEM
	Recessive (tt vs. TT/Tt)	0.84 (0.66, 1.08)	0.172	60.7	0.005	RME
*Apa*I	Allelic (A vs. a)	1.09 (0.80, 1.48)	0.594	91.5	0.000	RME
	Homozygous (AA vs. aa)	0.99 (0.59, 1.66)	0.973	85.1	0.000	RME
	Heterozygous (Aa vs. aa)	1.13 (0.71, 1.79)	0.600	88.9	0.000	REM
	Dominant (AA/Aa vs. aa)	1.10 (0.68, 1.80)	0.698	91.2	0.000	REM
	Recessive (AA vs. aa/Aa)	0.94 (0.71, 1.26)	0.700	72.0	0.000	RME
**MCI**						
*Fok*I	Allelic (f vs. F)	0.95 (0.75, 1.19)	0.646	0.0	0.775	FEM
	Homozygous (ff vs. FF)	0.87 (0.54, 1.43)	0.541	0.0	0.541	FEM
	Heterozygous (Ff vs. FF)	1.17 (0.80, 1.72)	0.423	0.0	0.937	FEM
	Dominant (ff/Ff vs. FF)	1.07 (0.74, 1.54)	0.706	0.0	0.866	FEM
	Recessive (ff vs. FF/Ff)	0.79 (0.54, 1.17)	0.241	0.0	0.823	FEM
*Bsm*I	Allelic (B vs. b)	0.56 (0.41, 0.75)	0.000*	20.9	0.282	FEM
	Homozygous (BB vs. bb)	0.40 (0.13, 1.19)	0.098	19.1	0.291	FEM
	Heterozygous (Bb vs. bb)	0.49 (0.32, 0.75)	0.001*	0.0	0.559	FEM
	Dominant (BB/Bb vs. bb)	0.48 (0.31, 0.73)	0.001*	10.2	0.328	FEM
	Recessive (BB vs. bb/Bb)	0.54 (0.33, 0.89)	0.015*	0.0	0.524	FEM
*Taq*I	Allelic (t vs. T)	1.19 (0.84, 1.70)	0.320	47.6	0.148	FEM
	Homozygous (tt vs. TT)	2.35 (0.92, 6.04)	0.076	45.3	0.161	FEM
	Heterozygous (Tt vs. TT)	0.93 (0.60, 1.44)	0.736	0.0	0.859	FEM
	Dominant (tt/Tt vs. TT)	1.04 (0.68, 1.59)	0.874	0.0	0.462	FEM
	Recessive (tt vs. TT/Tt)	2.41 (0.97, 6.00)	0.060	46.0	0.157	FME
*Apa*I	Allelic (A vs. a)	1.37 (1.12, 1.67)	0.002*	33.1	0.371	FME
	Homozygous (AA vs. aa)	1.92 (1.24, 2.97)	0.004*	23.5	0.270	FME
	Heterozygous (Aa vs. aa)	1.24 (0.92, 1.67)	0.154	0.0	0.685	FEM
	Dominant (AA/Aa vs. aa)	1.37 (1.03, 1.81)	0.028*	0.0	0.511	FEM
	Recessive (AA vs. aa/Aa)	1.72 (1.17, 2.52)	0.006*	29.8	0.234	FME

*P*, *P*-value of *Z*-test for statistical significance; *P*_*H*_, *P*-value of *Q*-test for heterogeneity test.

RETRACTED

*P < 0.05.

Stratification analyses of ethnicity displayed remarkable association between *Taq*I genotype and decreased AD risk among Caucasians (tt vs. TT: OR = 0.67, 95% CI = 0.49–0.93, *P* = 0.017). Likewise, the *Apa*I AA genotype evidently reduced the AD risk in Caucasian descents (A vs. a: OR = 0.75, 95% CI = 0.61–0.92, *P* = 0.006; AA vs. aa: OR = 0.60, 95% CI = 0.38–0.95, *P* = 0.028; AA vs. Aa/aa: OR = 0.63, 95% CI = 0.47–0.85, *P* = 0.003). When subgroup analyses were performed to assess the effect of heterogeneity on the results, the homozygous model of *Taq*I was significantly correlated with AD susceptibility in subgroups of PB (tt vs. TT: OR = 0.56, 95% CI = 0.34–0.93, *P* = 0.024), high quality score (tt vs. TT: OR = 0.67, 95% CI = 0.49–0.93, *P* = 0.017) and large sample size (tt vs. TT: OR = 0.56, 95% CI = 0.34–0.93, *P* = 0.024). In addition, the *Apa*I polymorphism was notably related to AD risk in PB (AA vs. aa: OR = 0.62, 95% CI = 0.42–0.91, *P* = 0.015), high quality score (A vs. a: OR = 0.82, 95% CI = 0.69–0.97, *P* = 0.023; AA vs. aa: OR = 0.60, 95% CI = 0.39–0.92, *P* = 0.020; AA vs. Aa/aa: OR = 0.63, 95% CI = 0.47–0.85, *P* = 0.003), and large sample size (AA vs. aa: OR = 0.62, 95% CI = 0.42–0.91, *P* = 0.015, Table 4). Except for the allelic, heterozygous and dominant models of VDR *Taq*I polymorphism, there was no heterogeneity in three other VDR gene polymorphisms.

**TABLE 4:** Meta-analysis results for the association between vitamin D receptor gene polymorphisms and AD based on subgroup analyses.

Locus	No.	Allele		Homozygote		Heterozygote		Dominant		Recessive	
		**OR (95% CI), *P***	***I*^2^ (%)**	**OR (95% CI), *P***	***I*^2^ (%)**	**OR (95% CI), *P***	***I*^2^ (%)**	**OR (95% CI), *P***	***I*^2^ (%)**	**OR (95% CI), *P***	***I*^2^ (%)**
**VDR *Fok*I polymorphism in AD**											
**Ethnicity**											
Caucasian	5	0.96 (0.83, 1.11), 0.593	0.0	1.05 (0.77, 1.43), 0.771	0.0	0.84 (0.68, 1.03), 0.099	0.0	0.88 (0.72, 1.07), 0.201	0.0	1.13 (0.84, 1.51), 0.415	0.0
Asian	1	1.24 (0.89, 1.15), 0.140	–	1.39 (0.76, 2.51), 0.283	–	1.56 (1.00, 2.43), 0.048	–	1.52 (1.00, 2.31), 0.053	–	1.07 (0.63, 1.81), 0.814	–
**Source of control**											
PB	1	1.24 (0.93, 1.64), 0.140	–	1.39 (0.76, 2.51), 0.283	–	1.56 (1.00, 2.43), 0.048	–	1.52 (1.00, 2.31), 0.053	–	0.86 (0.69, 1.08), 0.195	–
HB	5	0.96 (0.83, 1.10), 0.593	0.0	1.05 (0.77, 1.43), 0.771	0.0	0.84 (0.68, 1.03), 0.099	0.0	0.88 (0.72, 1.07), 0.201	0.0	1.01 (0.82, 1.26), 0.897	0.0
**NOS scores**											
N1	6	1.01 (0.89, 1.15), 0.850	0.0	1.11 (0.84, 1.46), 0.456	0.0	0.94 (0.78, 1.13), 0.525	38.5	0.97 (0.82, 1.16), 0.753	25.5	0.89 (0.76, 1.04), 0.131	0.0
**Sample size**											
S1	4	0.97 (0.76, 1.22), 0.766	0.0	1.10 (0.64, 1.89), 0.719	0.0	0.85 (0.61, 1.13), 0.333	0.0	0.89 (0.65, 1.22), 0.460	0.0	0.97 (0.78, 1.21), 0.796	0.0
S2	2	1.03 (0.89, 1.20), 0.676	54.4	1.11 (0.81, 1.53), 0.514	0.0	0.99 (0.79, 1.24), 0.912	82.4	1.01 (0.82, 1.25), 0.906	79.4	0.80 (0.66, 0.97), 0.021	0.0
**VDR BsmI polymorphism in AD**											
**Ethnicity**											
Caucasian	4	1.03 (0.82, 1.28), 0.824	0.0	1.02 (0.66, 1.56), 0.943	0.0	1.26 (0.88, 1.80), 0.210	0.0	1.16 (0.84, 1.61), 0.369	0.0	0.88 (0.60, 1.29), 0.501	40.4
Asian	1	1.22 (0.69, 2.17), 0.496	–	0.78 (0.03, 19.33), 0.881	–	1.31 (0.72, 2.39), 0.371	–	1.28 (0.70, 2.32), 0.422	–	0.76 (0.03, 18.71), 0.865	–
**Source of control**											
PB	1	1.22 (0.69, 2.17), 0.496	–	0.78 (0.03, 19.33), 0.881	–	1.31 (0.72, 2.39), 0.371	–	1.28 (0.70, 2.32), 0.422	–	0.76 (0.03, 18.71), 0.865	–
HB	4	1.03 (0.82, 1.28), 0.824	0.0	1.02 (0.66, 1.56), 0.943	0.0	1.26 (0.88, 1.80), 0.210	0.0	1.16 (0.84, 1.61), 0.369	0.0	0.88 (0.60, 1.29), 0.501	40.4
**NOS scores**											
N1	5	1.05 (0.85, 1.29), 0.655	0.0	1.01 (0.66, 1.54), 0.655	0.0	1.27 (0.94, 1.73), 0.125	0.0	1.19 (0.89, 1.58), 0.243	0.0	0.88 (0.60, 1.28), 0.491	20.6
**Sample size**											
S1	4	1.03 (0.82, 1.28), 0.824	0.0	1.02 (0.66, 1.56), 0.943	0.0	1.26 (0.88, 1.80), 0.210	0.0	1.16 (0.84, 1.61), 0.369	0.0	0.88 (0.60, 1.29), 0.501	40.4
S2	1	1.22 (0.69, 2.17), 0.496	–	0.78 (0.03, 19.33), 0.881	–	1.31 (0.72, 2.39), 0.371	–	1.28 (0.70, 2.32), 0.422	–	0.76 (0.03, 18.71), 0.865	–
**VDR TaqI polymorphism in AD**											
**Ethnicity**											
Caucasian	6	0.87 (0.65, 1.18), 0.373	67.4	0.67 (0.49, 0.93), 0.017*	51.8	0.85 (0.56, 1.27), 0.416	60.2	0.83 (0.54, 1.28), 0.402	68.1	0.78 (0.58, 1.05), 0.106	12.1
Asian	1	1.30 (0.73, 2.31), 0.380	–	0.79 (0.03, 19.46), 0.884	–	1.41 (0.77, 2.58), 0.270	–	1.36 (0.75, 2.49), 0.313	–	0.76 (0.03, 18.71), 0.865	–
**Source of control**											
PB	2	0.91 (0.52, 1.60), 0.741	70.1	0.56 (0.34, 0.93), 0.024*	0.0	0.88 (0.37, 2.08), 0.763	82.7	0.85 (0.37, 1.96), 0.716	82.7	0.77 (0.49, 1.20), 0.252	0.0
HB	5	0.93 (0.63, 1.39), 0.733	70.7	0.77 (0.50, 1.17), 0.221	57.9	0.95 (0.60, 1.51), 0.816	54.6	0.93 (0.56, 1.55), 0.776	66.8	0.79 (0.53, 1.18), 0.247	29.7
**NOS scores**											
N1	7	0.87 (0.65, 1.18), 0.534	65.9	0.67 (0.49, 0.93), 0.017*	42.2	0.91 (0.63, 1.34), 0.639	61.5	0.90 (0.60, 2.49), 0.584	68.1	0.78 (0.58, 1.05), 0.104	0.0
**Sample size**											
S1	5	0.93 (0.63, 1.39), 0.733	70.7	0.77 (0.50, 1.17), 0.221	57.9	0.95 (0.60, 1.51), 0.816	54.6	0.93 (0.56, 1.55), 0.776	66.8	0.79 (0.53, 1.18), 0.247	29.7
S2	2	0.91 (0.52, 1.60), 0.741	70.1	0.56 (0.34, 0.93), 0.024*	0.0	0.88 (0.37, 2.08), 0.763	82.7	0.85 (0.37, 1.96), 0.716	82.7	0.77 (0.49, 1.20), 0.252	0.0
**VDR ApaI polymorphism in AD**											
**Ethnicity**											
Caucasian	3	0.75 (0.61, 0.92), 0.006*	0.0	0.60 (0.38, 0.95), 0.028*	12.9	0.88 (0.58, 1.34), 0.553	60.7	0.75 (0.50, 1.12), 0.161	44.3	0.63 (0.47, 0.85), 0.003*	17.0
Asian	2	0.99 (0.79, 1.24), 0.917	0.0	0.81 (0.46, 1.43), 0.462	0.0	1.03 (0.74, 1.44), 0.865	0.0	1.01 (0.73, 1.39), 0.973	0.0	0.95 (0.61, 1.47), 0.806	0.0
**Source of control**											
PB	2	0.85 (0.72, 1.01), 0.065	42.0	0.62 (0.42, 0.91), 0.015*	0.0	0.91 (0.69, 1.19), 0.479	21.5	0.85 (0.66, 1.11), 0.236	42.4	0.76 (0.57, 1.01), 0.062	21.2
HB	3	0.82 (0.57, 1.17), 0.277	0.0	1.14 (0.44, 2.93), 0.792	0.0	2.00 (0.80, 4.97), 0.138	18.6	1.55 (0.63, 3.78), 0.337	0.0	0.61 (0.37, 0.99), 0.047	58.0
**NOS scores**											
N1	4	0.82 (0.69, 0.97), 0.023*	15.5	0.60 (0.39, 0.92), 0.020*	0.0	0.88 (0.58, 1.34), 0.553	49.3	0.75 (0.50, 1.12), 0.161	44.2	0.63 (0.47, 0.85), 0.003*	0.0
N2	1	0.96 (0.70, 1.32), 0.791	–	0.88 (0.46, 1.67), 0.695	–	1.03 (0.74, 1.44), 0.865	–	1.01 (0.73, 1.39), 0.973	–	0.95 (0.61, 1.47), 0.806	–
**Sample size**											
S1	2	0.82 (0.57, 1.17), 0.277	0.0	1.14 (0.44, 2.93), 0.792	0.0	2.00 (0.80, 4.97), 0.138	18.6	1.55 (0.63, 3.78), 0.337	0.0	0.61 (0.37, 0.99), 0.047	58.0
S2	3	0.85 (0.72, 1.01), 0.065	42.0	0.62 (0.42, 0.91), 0.015*	0.0	0.91 (0.69, 1.19), 0.479	21.5	0.85 (0.66, 1.11), 0.236	42.4	0.76 (0.57, 1.01), 0.062	21.2

*P < 0.05.

RETRACTED

### 3.4 Associations of VDR gene polymorphisms with PD risk

To identify the potential associations of VDR gene polymorphisms with the risk of PD, 12 studies about VDR *Fok*I polymorphism (2,979 cases and 3,484 controls), 11 studies about VDR *Bsm*I polymorphism (2,284 cases and 3,045 controls), 12 studies about *Taq*I polymorphism (3,001 cases and 3,566 controls), and 10 studies about VDR *Apa*I polymorphism (2,284 cases and 2,930 controls) were included in this meta-analysis, respectively. As shown in Table 3, there were no associations between *Fok*I (f vs. F: OR = 0.94, 95% CI = 0.79–1.11, *P* = 0.474; ff vs. FF: OR = 0.84, 95% CI = 0.59–1.21, *P* = 0.355; Ff vs. FF: OR = 1.10, 95% CI = 0.83–2.36, *P* = 0.505; ff/Ff vs. FF: OR = 1.00, 95% CI = 0.81–1.24, *P* = 0.999; ff vs. Ff/FF: OR = 0.81, 95% CI = 0.56–1.16, *P* = 0.252, Supplementary Figure 4), *Bsm*I (B vs. b: OR = 1.06, 95% CI = 0.97–1.16, *P* = 0.231; BB vs. bb: OR = 1.08, 95% CI = 0.89–1.30, *P* = 0.437; Bb vs. bb: OR = 1.14, 95% CI = 0.96–1.36, *P* = 0.070; BB/Bb vs. bb: OR = 1.13, 95% CI = 0.99–1.29, *P* = 0.208; BB vs. Bb/bb: OR = 1.00, 95% CI = 0.85–1.17, *P* = 0.992, Supplementary Figure 5), and *Apa*I (A vs. a: OR = 1.09, 95% CI = 0.80–1.48, *P* = 0.594; AA vs. aa: OR = 0.99, 95% CI = 0.59–1.66, *P* = 0.973; Aa vs. aa: OR = 1.13, 95% CI = 0.71–1.79, *P* = 0.600; AA/Aa vs. aa: OR = 1.10, 95% CI = 0.68–1.80, *P* = 0.698; AA vs. Aa/aa: OR = 0.94, 95% CI = 0.71–1.26, *P* = 0.700, Supplementary Figure 6) gene polymorphisms and the risk of PD. Intriguingly, the dominant model of *Taq*I polymorphism was slightly linked with elevated PD susceptibility (tt/Tt vs. TT: OR = 1.12, 95% CI = 0.97–1.29, *P* = 0.035, Figure 3).

RETRACTED

**FIGURE 3:** Forest plots for the association between VDR *Taq*I polymorphism and PD risk in five models. **(A)** Allele model; **(B)** homozygote model; **(C)** heterozygote model; **(D)** dominant model; **(E)** recessive model.

As revealed by ethnicity subgroup analysis, there was no significant relationships between *Fok*I, *Bsm*I, and *Apa*I gene polymorphisms and PD susceptibility in Table 5. Conversely, the *Taq*I polymorphism slightly increased the risk of PD in heterozygous models among Asians (Tt vs. TT: OR = 1.22, 95% CI = 1.00–1.49, *P* = 0.047). When stratified by source of control, quality scores, and sample size, the *Fok*I variant was definitely associated with PD susceptibility in the HB (f vs. F: OR = 0.80, 95% CI = 0.68–0.93, *P* = 0.003; ff vs. FF: OR = 0.59, 95% CI = 0.45–0.77, *P* = 0.000; ff/Ff vs. FF: OR = 0.58, 95% CI = 0.44–0.76, *P* = 0.000), low quality score (f vs. F: OR = 0.82, 95% CI = 0.73–0.92, *P* = 0.001; ff vs. FF: OR = 0.63, 95% CI = 0.50–0.78, *P* = 0.000; ff/Ff vs. FF: OR = 0.58, 95% CI = 0.45–0.81, *P* = 0.001), high quality score (ff/Ff vs. FF: OR = 1.50, 95% CI = 1.16–1.93, *P* = 0.002), and small sample size (f vs. F: OR = 0.55, 95% CI = 0.38–0.80, *P* = 0.002; ff vs. FF: OR = 0.32, 95% CI = 0.15–0.78, *P* = 0.003; ff/Ff vs. FF: OR = 0.37, 95% CI = 0.21–0.65, *P* = 0.001). There was a significant relation between VDR *Apa*I variant and PD predisposition in the PB subgroup (A vs. a: OR = 0.85, 95% CI = 0.75–0.95, *P* = 0.005; AA vs. aa: OR = 0.70, 95% CI = 0.56–0.89, *P* = 0.003; AA/Aa vs. aa: OR = 0.80, 95% CI = 0.66–0.98, *P* = 0.027; AA vs. Aa/aa: OR = 0.77, 95% CI = 0.59–1.01, *P* = 0.058, Table 5). Stratified analyses by source of control, quality score and sample size, no prominent relationships between the *Bsm*I and *Taq*I polymorphisms and PD risk was detected. For the *Fok*I, heterogeneity was shown to present in all five comparisons of overall, and Caucasian subgroup. In addition, the heterogeneity existed in overall group and Asian subgroup of the *Taq*I. However, we discovered no heterogeneity in the *Bsm*I and *Apa*I polymorphisms.

**TABLE 5:** Meta-analysis results for the association between vitamin D receptor gene polymorphisms and PD based on subgroup analyses.

Locus	No.	Allele		Homozygote		Heterozygote		Dominant		Recessive	
		**OR (95% CI), *P***	***I*^2^** **(%)**	**OR (95% CI), *P***	***I*^2^** **(%)**	**OR (95% CI), *P***	***I*^2^ (%)**	**OR (95% CI), *P***	***I*^2^ (%)**	**OR (95% CI), *P***	***I*^2^ (%)**
**VDR *Fok*I polymorphism in PD**											
**Ethnicity**											
Caucasian	5	0.96 (0.73, 1.27), 0.767	83.8	0.84 (0.47, 1.51), 0.567	84.6	1.40 (0.83, 2.36), 0.213	88.8	1.13 (0.79, 1.61), 0.513	80.3	0.73 (0.40, 1.34), 0.312	88.0
Asian	7	0.88 (0.70, 1.10), 0.443	74.1	0.77 (0.46, 1.27), 0.303	76.8	0.91 (0.78, 1.07), 0.250	0.0	0.90 (0.76, 1.08), 0.256	24.1	0.78 (0.48, 1.27), 0.317	80.9
**Source of control**											
PB	5	1.09 (0.89, 1.35), 0.405	78.6	1.20 (0.79, 1.83), 0.402	76.8	1.05 (0.83, 1.33), 0.666	57.6	1.09 (0.83, 1.42), 0.530	71.2	1.19 (0.86, 1.66), 0.292	69.0
HB	7	0.80 (0.68, 0.93), 0.003*	34.3	0.59 (0.45, 0.77), 0.000*	10.9	1.15 (0.72, 1.85), 0.522	83.8	0.91 (0.69, 1.22), 0.590	63.2	0.52 (0.37, 0.72), 0.000*	46.6
**NOS scores**											
N1	9	0.82 (0.73, 0.92), 0.001*	17.1	0.63 (0.50, 0.78), 0.000*	0.0	1.08 (0.76, 1.53), 0.656	78.7	0.91 (0.73, 1.12), 0.354	51.4	0.58 (0.44, 0.76), 0.000*	45.5
N2	3	1.24 (0.99, 1.55), 0.058	75.6	1.57 (1.06, 2.33), 0.024	66.9	1.12 (0.81, 1.56), 0.498	73.4	1.23 (0.88, 1.72), 0.234	77.0	1.50 (1.16, 1.93), 0.002*	36.4
**Sample size**											
S1	2	0.55 (0.38, 0.80), 0.002*	9.1	0.32 (0.15, 0.68), 0.003*	0.0	0.80 (0.45, 1.41), 0.439	0.0	0.61 (0.36, 1.04), 0.071	0.0	0.37 (0.21, 0.65), 0.001*	0.0
S2	10	0.98 (0.84, 1.15), 0.819	75.9	0.91 (0.64, 1.31), 0.609	79.5	1.12 (0.86, 1.47), 0.391	80.2	1.04 (0.85, 1.27), 0.707	70.5	0.87 (0.60, 1.25), 0.437	83.4
**VDR BsmI polymorphism in PD**											
**Ethnicity**											
Caucasian	6	1.05 (0.94, 1.17), 0.389	0.0	1.06 (0.85, 1.32), 0.597	0.0	1.15 (0.96, 1.36), 0.122	15.4	1.12 (0.95, 1.32), 0.166	0.8	0.99 (0.82, 1.20), 0.897	0.0
Asian	5	1.04 (0.89, 1.22), 0.630	18.5	1.16 (0.82, 1.63), 0.397	0.0	1.14 (0.87, 1.48), 0.343	38.2	1.02 (0.82, 1.27), 0.47	34.3	1.08 (0.83, 1.40), 0.575	0.0
**Source of control**											
PB	3	1.09 (0.95, 1.24), 0.214	0.0	1.13 (0.87, 1.47), 0.368	0.0	1.22 (0.99, 1.51), 0.057	0.0	1.19 (0.98, 1.45), 0.076	0.0	1.01 (0.80, 1.27), 0.965	0.0
HB	8	1.01 (0.90, 1.14), 0.854	0.0	1.05 (0.81, 1.36), 0.702	0.0	0.99 (0.81, 1.19), 0.874	29.5	1.00 (0.84, 1.20), 0.972	18.1	11.03 (0.84, 1.27), 0.787	0.0
**NOS scores**											
N1	8	1.02 (0.89, 1.16), 0.795	0.0	1.06 (0.80, 1.39), 0.697	0.0	1.02 (0.83, 1.24), 0.876	22.4	1.03 (0.85, 1.24), 0.783	11.9	1.01 (0.81, 1.26), 0.911	0.0
N2	3	1.07 (0.95, 1.21), 0.268	0.0	1.11 (0.87, 1.42), 0.389	0.0	1.16 (0.95, 1.41), 0.136	48.5	1.15 (0.95, 1.38), 0.147	42.1	1.02 (0.82, 1.27), 0.830	0.0
**Sample size**											
S1	2	1.06 (0.77, 1.45), 0.905	0.0	1.08 (0.57, 2.06), 0.813	0.0	0.89 (0.50, 1.56), 0.673	0.0	0.95 (0.56, 1.62), 0.841	0.0	1.21 (0.74, 1.97), 0.458	0.0
S2	9	1.05 (0.95, 1.15), 0.207	0.0	1.09 (0.90, 1.32), 0.384	0.0	1.10 (0.95, 1.27), 0.186	38.2	1.10 (0.96, 1.25), 0.187	30.4	1.00 (0.85, 1.18), 0.998	0.0
**VDR TaqI polymorphism in PD**											
**Ethnicity**											
Caucasian	6	1.00 (0.91, 1.11), 0.997	65.5	0.94 (0.76, 1.15), 0.540	65.4	1.26 (0.86, 1.87), 0.239	82.3	1.12 (0.97, 1.29), 0.138	65.6	0.83 (0.54, 1.29), 0.408	79.4
Asian	6	1.01 (0.88, 1.15), 0.916	0.0	1.00 (0.72, 1.39), 0.997	0.0	1.22 (1.00, 1.49), 0.047*	0.0	1.17 (0.96, 1.41), 0.114	0.0	0.83 (0.66, 1.03), 0.095	0.0
**Source of control**											
PB	5	1.04 (0.93, 1.15), 0.539	56.3	1.04 (0.82, 1.32), 0.739	55.1	1.13 (0.87, 1.47), 0.373	58.8	1.11 (0.95, 1.29), 0.201	64.3	0.95 (0.77, 1.16), 0.599	0.0
HB	7	0.97 (0.86, 1.09), 0.557	5.7	0.86 (0.67, 1.12), 0.263	13.7	1.34 (0.93, 1.91), 0.113	68.0	1.17 (0.98, 1.40), 0.079	0.0	0.80 (0.54, 1.20), 0.284	70.2
**NOS scores**											
N1	9	0.94 (0.85, 1.04), 0.218	18.2	0.81 (0.64, 1.02), 0.070	16.5	1.29 (0.95, 1.74), 0.104	68.4	1.10 (0.95, 1.28), 0.213	24.1	0.75 (0.55, 1.02), 0.067	61.0
N2	3	1.11 (0.98, 1.25), 0.114	18.5	1.19 (0.92, 1.56), 0.191	0.0	1.15 (0.84, 1.58), 0.376	58.5	1.19 (0.99, 1.43), 0.065	56.4	1.08 (0.85, 1.37), 0.538	0.0
**Sample size**											
S1	3	1.14 (0.89, 1.47), 0.296	0.0	1.23 (0.62, 2.47), 0.557	0.0	1.15 (0.83, 1.61), 0.397	0.0	1.17 (0.85, 1.62), 0.343	0.0	1.18 (0.70, 2.01), 0.529	0.0
S2	9	0.99 (0.91, 1.07), 0.779	45.7	0.94 (0.78, 1.13), 0.494	41.6	1.26 (0.97, 1.65), 0.082	72.4	1.13 (1.00, 1.28), 0.054	44.7	0.80 (0.61, 1.05), 0.111	66.1
**VDR ApaI polymorphism in PD**											
**Ethnicity**											
Caucasian	5	0.91 (0.80, 1.03), 0.137	26.9	0.82 (0.62, 1.08), 0.163	34.9	0.92 (0.75, 1.12), 0.378	8.3	0.88 (0.73, 1.06), 0.171	9.6	0.87 (0.69, 1.10), 0.236	43.8
Asian	5	1.26 (0.59, 2.71), 0.556	95.8	1.10 (0.22, 5.52), 0.905	93.6	1.18 (0.42, 3.33), 0.751	94.2	1.15 (0.38, 3.53), 0.806	95.4	1.21 (0.52, 2.84), 0.054	86.2
**Source of control**											
PB	3	0.85 (0.75, 0.95), 0.005*	0.0	0.70 (0.56, 0.89), 0.003*	0.0	0.86 (0.69, 1.09), 0.211	19.5	0.80 (0.66, 0.98), 0.027*	0.0	0.77 (0.59, 1.01), 0.058	47.0
HB	7	1.23 (0.73, 2.07), 0.439	93.7	1.21 (0.46, 3.17), 0.695	89.5	1.22 (0.58, 2.57), 0.594	91.3	1.21 (0.55, 2.69), 0.634	93.1	1.16 (0.70, 1.92), 0.576	78.5
**NOS scores**											
N1	7	1.18 (0.71, 1.95), 0.525	93.9	1.10 (0.44, 2.76), 0.845	89.7	1.20 (0.58, 2.46), 0.742	91.5	1.16 (0.53, 2.53), 0.707	93.4	1.05 (0.65, 1.69), 0.839	78.3
N2	3	0.90 (0.76, 1.06), 0.197	42.3	0.79 (0.54, 1.14), 0.205	49.8	0.89 (0.67, 1.19), 0.442	38.8	0.85 (0.67, 1.09), 0.210	29.4	0.86 (0.60, 1.23), 0.399	64.6
**Sample size**											
S1	2	0.82 (0.38, 1.75), 0.600	81.0	0.43 (0.04, 5.37), 0.516	86.9	0.46 (0.05, 4.42), 0.504	85.2	0.46 (0.04, 4.81), 0.513	87.1	0.90 (0.48, 1.68), 0.743	38.7
S2	8	1.16 (0.82, 1.64), 0.407	93.1	1.10 (0.63, 1.92), 0.732	87.1	1.26 (0.77, 2.07), 0.354	90.5	1.24 (0.73, 2.10), 0.431	92.6	0.97 (0.69, 1.36), 0.843	77.6

*P < 0.05.

RETRACTED

### 3.5 Associations of VDR gene polymorphisms with MCI risk

In general, three eligible studies with 329 cases and 320 controls for *Fok*I, three studies with 400 cases and 319 controls for *Bsm*I, three studies with 404 cases and 252 controls for *Taq*I, and four studies with 528 cases and 385 controls for *Apa*I were finally included in our study. As regards *Fok*I polymorphism, the variant genotypes had no significant association with MCI risk in the five genetic models (f vs. F: OR = 0.95, 95% CI = 0.75–1.19, *P* = 0.646; ff vs. FF: OR = 0.87, 95% CI = 0.54–1.43, *P* = 0.541; Ff vs. FF: OR = 1.17, 95% CI = 0.80–1.72, *P* = 0.001; Ff vs. FF: OR = 1.17, 95% CI = 0.80–1.72, *P* = 0.001; ff/Ff vs. FF: OR = 1.07, 95% CI = 0.74–1.54, *P* = 0.706; ff vs. FF/Ff: OR = 0.79, 95% CI = 0.54–1.17, *P* = 0.241, Supplementary Figure 7). The integrated analyses demonstrated that VDR *Bsm*I polymorphism was evidently correlated with susceptibility to MCI (B vs. b: OR = 0.56, 95% CI = 0.41–0.75, *P* = 0.000; Bb vs. bb: OR = 0.49, 95% CI = 0.32–0.75, *P* = 0.001; BB/Bb vs. bb: OR = 0.48, 95% CI = 0.31–0.73, *P* = 0.001; BB vs. Bb/bb: OR = 0.54, 95% CI = 0.33–0.89, *P* = 0.015, Figure 4). No clear correlation was found between the *Taq*I variant and MCI susceptibility (t vs. T: OR = 1.19, 95% CI = 0.84–1.70, *P* = 0.320; tt vs. TT: OR = 2.35, 95% CI = 0.92–6.04, *P* = 0.076; Tt vs. TT: OR = 0.93, 95% CI = 0.60–1.44, *P* = 0.736; tt/Tt vs. TT: OR = 1.04, 95% CI = 0.68–1.59, *P* = 0.874; tt vs. TT/Tt: OR = 2.41, 95% CI = 0.97–6.00, *P* = 0.060, Supplementary Figure 8). A statistically significant association of VDR *Apa*I polymorphism with overall PD risk was discovered in allelic, homozygous, dominant, and recessive models (A vs. a: OR = 1.37, 95% CI = 1.12–1.67, *P* = 0.002; AA vs. aa: OR = 1.92, 95% CI = 1.24–2.97, *P* = 0.004; AA/Aa vs. aa: OR = 1.37, 95% CI = 1.03–1.81, *P* = 0.028; AA vs. Aa/aa: OR = 1.72, 95% CI = 1.17–2.52, *P* = 0.006, Figure 5 and Table 6).

**FIGURE 4:** Forest plots for the association between VDR *Bsm*I polymorphism and MCI risk in five models. **(A)** Allele model; **(B)** homozygote model; **(C)** heterozygote model; **(D)** dominant model; **(E)** recessive model.

RETRACTED

**FIGURE 5:** Forest plots for the association between VDR *Apa*I polymorphism and MCI risk in five models. **(A)** Allele model; **(B)** homozygote model; **(C)** heterozygote model; **(D)** dominant model; **(E)**: recessive model.

**TABLE 6:** Meta-analysis results for the association between vitamin D receptor gene polymorphisms and MCI based on subgroup analyses.

Locus	No.	Allele		Homozygote		Heterozygote		Dominant		Recessive	
		**OR (95% CI), *P***	***I*^2^ (%)**	**OR (95% CI), *P***	***I*^2^ (%)**	**OR (95% CI), *P***	***I*^2^ (%)**	**OR (95% CI), *P***	***I*^2^ (%)**	**OR (95% CI), *P***	***I*^2^ (%)**
**VDR *Fok*I polymorphism in MCI**											
**Ethnicity**											
Caucasian	2	1.00 (0.66, 1.51), 0.987	0.0	0.98 (0.42, 2.27), 0.956	0.0	1.18 (0.57, 2.44), 0.648	0.0	1.12 (0.57, 2.20), 0.747	0.0	0.90 (0.47, 1.71), 0.738	0.0
Asian	1	0.93 (0.71, 1.22), 0.591	–	0.82 (0.47, 1.43), 0.487	–	1.16 (0.74, 1.83), 0.510	–	1.05 (0.69, 1.62), 0.809	–	0.74 (0.46, 1.20), 0.223	–
**Source of control**											
PB	1	0.93 (0.71, 1.22), 0.591	–	0.82 (0.47, 1.43), 0.487	–	1.16 (0.74, 1.83), 0.510	–	1.05 (0.69, 1.62), 0.809	–	0.74 (0.46, 1.20), 0.223	–
HB	2	1.00 (0.66, 1.51), 0.987	0.0	0.98 (0.42, 2.27), 0.956	0.0	1.18 (0.57, 2.44), 0.648	0.0	1.12 (0.57, 2.20), 0.747	0.0	0.90 (0.47, 1.71), 0.738	0.0
**NOS scores**											
N1	2	1.00 (0.66, 1.51), 0.987	0.0	0.98 (0.42, 2.27), 0.956	0.0	1.18 (0.57, 2.44), 0.648	0.0	1.12 (0.57, 2.20), 0.747	0.0	0.90 (0.47, 1.71), 0.738	0.0
N2	1	0.93 (0.71, 1.22), 0.591	–	0.82 (0.47, 1.43), 0.487	–	1.16 (0.74, 1.83), 0.510	–	1.05 (0.69, 1.62), 0.809	–	0.74 (0.46, 1.20), 0.223	–
**Sample size**											
S1	2	1.00 (0.66, 1.51), 0.987	0.0	0.98 (0.42, 2.27), 0.956	0.0	1.18 (0.57, 2.44), 0.648	0.0	1.12 (0.57, 2.20), 0.747	0.0	0.90 (0.47, 1.71), 0.738	0.0
S2	1	0.93 (0.71, 1.22), 0.591	–	0.82 (0.47, 1.43), 0.487	–	1.16 (0.74, 1.83), 0.510	–	1.05 (0.69, 1.62), 0.809	–	0.74 (0.46, 1.20), 0.223	–
**VDR BsmI polymorphism in MCI**											
**Ethnicity**											
Caucasian	1	1.16 (0.45, 3.01), 0.763	–	1.67 (0.18, 15.13), 0.650	–	0.97 (0.25, 3.85), 0.968	–	1.07 (0.29, 3.99), 0.918	–	1.69 (0.21, 13.50), 0.619	–
Asian	2	0.51 (0.37, 0.70), 0.000*	0.0	0.24 (0.06, 0.92), 0.038*	0.0	0.45 (0.29, 0.71), 0.001*	0.0	0.43 (0.28, 0.68), 0.000*	0.0	0.50 (0.30, 0.84), 0.008*	0.0
**Source of control**											
PB	1	0.51 (0.37, 0.70), 0.000*	0.0	0.24 (0.06, 0.92), 0.038*	0.0	0.45 (0.29, 0.71), 0.001*	0.0	0.43 (0.28, 0.68), 0.000*	0.0	0.50 (0.30, 0.84), 0.008*	0.0
HB	2	1.16 (0.45, 3.01), 0.763	–	1.67 (0.18, 15.13), 0.650	–	0.97 (0.25, 3.85), 0.968	–	1.07 (0.29, 3.99), 0.918	–	1.69 (0.21, 13.50), 0.619	–
**NOS scores**											
N1	2	0.60 (0.40, 0.90), 0.013*	55.8	0.38 (0.11, 1.24), 0.109	58.8	0.61 (0.22, 1.68), 0.338	0.0	0.53 (0.21, 1.37), 0.192	52.4	0.53 (0.32, 0.89), 0.015*	21.4
N2	1	0.51 (0.33, 0.79), 0.003*	–	0.56 (0.04, 8.98), 0.680	–	0.46 (0.29, 0.75), 0.002*	–	0.46 (0.29, 0.75), 0.001*	–	0.65 (0.04, 10.52), 0.764	–
**Sample size**											
S1	2	0.60 (0.40, 0.90), 0.013*	55.8	0.38 (0.11, 1.24), 0.109	58.8	0.61 (0.22, 1.68), 0.338	0.0	0.53 (0.21, 1.37), 0.192	52.4	0.53 (0.32, 0.89), 0.015*	21.4
S2	1	0.51 (0.33, 0.79), 0.003*	–	0.56 (0.04, 8.98), 0.680	–	0.46 (0.29, 0.75), 0.002*	–	0.46 (0.29, 0.75), 0.001*	–	0.65 (0.04, 10.52), 0.764	–
**VDR TaqI polymorphism in MCI**											
**Ethnicity**											
Caucasian	2	1.46 (0.96, 2.23), 0.074	0.0	3.23 (1.11, 9.40), 0.031*	23.1	1.03 (0.58, 1.83), 0.926	0.0	1.28 (0.74, 2.22), 0.386	0.0	3.20 (1.14, 8.94), 0.027*	29.0
Asian	1	0.72 (0.37, 1.38), 0.317	–	0.21 (0.01, 5.27), 0.345	–	0.80 (0.40, 1.59), 0.522	–	0.75 (0.38, 1.48), 0.406	–	0.22 (0.01, 5.37), 0.351	–
**Source of control**											
PB	1	0.72 (0.37, 1.38), 0.317	–	0.21 (0.01, 5.27), 0.345	–	0.80 (0.40, 1.59), 0.522	–	0.75 (0.38, 1.48), 0.406	–	0.22 (0.01, 5.37), 0.351	–
HB	2	1.46 (0.96, 2.23), 0.074	0.0	3.23 (1.11, 9.40), 0.031*	23.1	1.03 (0.58, 1.83), 0.926	0.0	1.28 (0.74, 2.22), 0.386	0.0	3.20 (1.14, 8.94), 0.027*	29.0
**NOS scores**											
N1	2	1.46 (0.96, 2.23), 0.074	0.0	3.23 (1.11, 9.40), 0.031*	23.1	1.03 (0.58, 1.83), 0.926	0.0	1.28 (0.74, 2.22), 0.386	0.0	3.20 (1.14, 8.94), 0.027*	29.0
N2	1	0.72 (0.37, 1.38), 0.317	–	0.21 (0.01, 5.27), 0.345	–	0.80 (0.40, 1.59), 0.522	–	0.75 (0.38, 1.48), 0.406	–	0.22 (0.01, 5.37), 0.351	–
**Sample size**											
S1	2	1.46 (0.96, 2.23), 0.074	0.0	3.23 (1.11, 9.40), 0.031*	23.1	1.03 (0.58, 1.83), 0.926	0.0	1.28 (0.74, 2.22), 0.386	0.0	3.20 (1.14, 8.94), 0.027*	29.0
S2	1	0.72 (0.37, 1.38), 0.317	–	0.21 (0.01, 5.27), 0.345	–	0.80 (0.40, 1.59), 0.522	–	0.75 (0.38, 1.48), 0.406	–	0.22 (0.01, 5.37), 0.351	–
**VDR ApaI polymorphism in MCI**											
**Ethnicity**											
Caucasian	2	1.62 (1.10, 2.38), 0.016*	0.0	2.63 (1.18, 5.87), 0.018*	0.0	1.03 (0.53, 2.01), 0.934	0.0	1.46 (0.79, 2.73), 0.228	0.0	2.28 (1.21, 4.30), 0.011*	39.7
Asian	2	1.28 (1.02, 1.62), 0.036*	63.6	1.67 (0.99, 2.82), 0.056	63.9	1.30 (0.93, 1.81), 0.121	8.2	1.35 (0.98, 1.84), 0.064	55.3	1.44 (0.89, 2.35), 0.142	30.3
**Source of control**											
PB	2	1.28 (1.02, 1.62), 0.036*	63.6	1.67 (0.99, 2.82), 0.056	63.9	1.30 (0.93, 1.81), 0.121	8.2	1.35 (0.98, 1.84), 0.064	0.0	1.44 (0.89, 2.35), 0.142	39.7
HB	2	1.62 (1.10, 2.38), 0.016*	0.0	2.63 (1.18, 5.87), 0.018*	0.0	1.03 (0.53, 2.01), 0.934	0.0	1.46 (0.79, 2.73), 0.228	55.3	2.28 (1.21, 4.30), 0.011*	30.3
**NOS scores**											
N1	3	1.62 (1.24, 2.10), 0.000*	0.0	2.63 (1.18, 5.87), 0.018*	0.0	1.03 (0.53, 2.01), 0.934	0.0	1.46 (0.79, 2.73), 0.228	0.0	2.28 (1.21, 4.30), 0.011*	0.0
N2	1	1.08 (0.80, 1.47), 0.613	–	1.67 (0.99, 2.82), 0.056	–	1.30 (0.93, 1.81), 0.121	–	1.35 (0.98, 1.84), 0.064	–	1.44 (0.89, 2.35), 0.142	–
**Sample size**											
S1	3	1.62 (1.24, 2.10), 0.000*	0.0	2.62 (1.52, 4.53), 0.001*	0.0	1.36 (0.88, 2.09), 0.164	0.0	1.69 (1.13, 2.54), 0.011*	0.0	2.11 (1.33, 3.32), 0.772	0.0
S2	1	1.08 (0.80, 1.47), 0.613	–	1.07 (0.51, 2.25), 0.865	–	1.15 (0.76, 1.72), 0.516	–	1.13 (0.77, 1.67), 0.532	–	1.01 (0.49, 2.09), 0.982	–

*P < 0.05.

RETRACTED

To further elucidate whether the potential underestimation of the true effect on MCI risk, we stratified these studies in the light of ethnicity, source of controls, quality scores, and sample size. As shown in Table 6, the *Fok*I and *Taq*I polymorphisms were not remarkably linked with MCI risk. Interestingly, carriers with the BB genotype seemed to have a stronger association with low MCI risk among Asians (B vs. b: OR = 0.51, 95% CI = 0.37–0.70, *P* = 0.000; BB vs. bb: OR = 0.24, 95% CI = 0.06–0.92, *P* = 0.038; Bb vs. bb: OR = 0.45, 95% CI = 0.29–0.71, *P* = 0.001; BB/Bb vs. bb: OR = 0.43, 95% CI = 0.28–0.68, *P* = 0.000; BB vs. Bb/bb: OR = 0.50, 95% CI = 0.30–0.84, *P* = 0.008). There were remarkable associations between *Bsm*I polymorphism and MCI risk in PB, small sample size, large sample size, low quality score (B vs. b: OR = 0.60, 95% CI = 0.40–0.90, *P* = 0.013; BB vs. Bb/bb: OR = 0.53, 95% CI = 0.32–0.89, *P* = 0.015), high quality score (B vs. b: OR = 0.51, 95% CI = 0.33–0.79, *P* = 0.003; Bb vs. bb: OR = 0.46, 95% CI = 0.29–0.75, *P* = 0.002; BB/Bb vs. bb: OR = 0.46, 95% CI = 0.29–0.75, *P* = 0.001). Next, stratified analyses showed that the *Apa*I variant was positively associated with the predisposition to MCI in Caucasian (A vs. a: OR = 1.62, 95% CI = 1.10–2.38, *P* = 0.016; AA vs. aa: OR = 2.63, 95% CI = 1.18–5.87, *P* = 0.018; AA vs. Aa/aa: OR = 2.28, 95% CI = 1.21–4.30, *P* = 0.011) and Asian descents (A vs. a: OR = 1.28, 95% CI = 1.02–1.62, *P* = 0.036). Similarly, a prominent correlation of the *Apa*I polymorphism and MCI risk was discovered in subgroups of HB (A vs. a: OR = 1.62, 95% CI = 1.10–2.38, *P* = 0.016; AA vs. aa: OR = 2.63, 95% CI = 1.18–5.87, *P* = 0.018; AA vs. Aa/aa: OR = 2.28, 95% CI = 1.21–4.30, *P* = 0.011), PB (A vs. a: OR = 1.28, 95% CI = 1.02–1.62, *P* = 0.036), low quality score, and small sample size (A vs. a: OR = 1.62, 95% CI = 1.24–2.10, *P* = 0.000; AA vs. aa: OR = 2.62, 95% CI = 1.52–4.53, *P* = 0.001; AA/Aa vs. aa: OR = 1.69, 95% CI = 1.13–2.54, *P* = 0.011, Table 6). The result of heterogeneity test exhibited *I*^2^ < 50%, indicating no heterogeneity in all the five genetic models of these VDR SNPs, and thus fixed-effects model was used to examine the correlation.

RETRACTED

### 3.6 Sensitivity analysis and publication bias

Sensitivity analysis was conducted to estimate the effect of the respective study on the pooled ORs. No individual study dramatically influence the combined ORs under any genetic models, indicating that the results were relatively reliable and stable (Figure 6 and Supplementary Figures 9, 10). Funnel plots were found to be symmetrical for all genetic models. Besides, publication bias was evaluated by Begg’s funnel plot analysis (Supplementary Figure 11) and Egger’s test (Figure 7 and Table 7). As shown in Table 7, no statistically significant publication bias was observed for the correlation of four VDR gene polymorphisms with AD and MCI susceptibility. As regards PD risk, Egger’s tests showed no publication bias except for homologous and recessive models of *Fok*I polymorphism (ff vs. FF: *P*_*E*_ = 0.019; ff vs. FF/Ff: *P_*E*_* = 0.007).

**FIGURE 6:** Sensitivity analysis for VDR gene polymorphism and PD risk in dominant model. **(A)** *Fok*I polymorphism; **(B)**: *Bsm*I polymorphism; **(C)** *Taq*I polymorphism; **(D)** *Apa*I polymorphism.

**FIGURE 7:** Egger’s linear regression plot for detecting the publication bias in the dominant model of VDR SNPs. **(A)** *Fok*I polymorphism and AD risk; **(B)** *Bsm*I polymorphism and AD risk; **(C)** *Taq*I polymorphism and AD risk; **(D)** *Apa*I polymorphism and AD risk; **(E)** *Fok*I polymorphism and PD risk; **(F)** *Bsm*I polymorphism and PD risk; **(G)** *Taq*I polymorphism and PD risk; **(H)** *Apa*I polymorphism and PD risk; **(I)** *Fok*I polymorphism and MCI risk; **(J)** *Bsm*I polymorphism and MCI risk; **(K)** *Taq*I polymorphism and MCI risk; **(L)** *Apa*I polymorphism and MCI risk.

**TABLE 7:** Publication bias of the five genetic models for multiple VDR SNPs in AD, MCI, and PD.

Variables	Allelic		Homozygous		Heterozygous		Dominant		Recessive	
	***P*_*B*_**	***P*_*E*_**	***P*_*B*_**	***P*_*E*_**	***P*_*B*_**	***P*_*E*_**	***P*_*B*_**	***P*_*E*_**	***P*_*B*_**	***P*_*E*_**
**AD**										
*Fok*I	0.091	0.248	0.348	0.311	0.188	0.195	0.188	0.193	0.348	0.363
*Bsm*I	0.327	0.094	0.624	0.440	1.000	0.325	1.000	0.274	0.624	0.449
*Taq*I	0.293	0.166	0.548	0.303	0.652	0.252	0.652	0.224	0.293	0.305
*Apa*I	0.624	0.404	0.624	0.349	0.624	0.918	0.624	0.946	0.624	0.259
**PD**										
*Fok*I	0.075	0.085	0.006s*	0.019*	0.273	0.243	0.217	0.179	0.006*	0.007*
*Bsm*I	0.052	0.062	0.139	0.104	0.036*	0.057	0.036*	0.069	0.243	0.515
*Taq*I	0.411	0.624	0.484	0.707	0.583	0.888	0.493	0.839	0.586	0.547
*Apa*I	0.245	0.244	0.144	0.217	0.060	0.485	0.060	0.487	0.251	0.135
**MCI**										
*Fok*I	0.117	0.288	0.117	0.209	0.117	0.386	0.117	0.366	0.117	0.136
*Bsm*I	0.177	0.011*	0.602	0.798	0.602	0.554	0.602	0.562	0.602	0.553
*Taq*I	0.602	0.593	0.296	0.058	0.602	0.876	0.602	0.843	0.117	0.096
*Apa*I	0.497	0.903	0.497	0.876	0.497	0.676	0.497	0.688	1.000	0.582

*P*_*B*_, *P*-value of Begg’s rank correlation test; *P*_*E*_, *P*-value of Egger’s linear regression test.

RETRACTED

*P < 0.05.

### 3.7 FPRP results

We explored determinants of FPRP across a range of probabilities to determine whether a given association of VDR SNPs with AD, PD, and MCI risk is deserving of attention or is noteworthy. In this respect, we detected that our main results were further supported by FPRP analysis. As shown in Table 8, with a prior probability <0.20, VDR *Taq*I and *Apa*I polymorphisms were significantly associated with the risk of AD. Similarly, with a prior probability of 0.20, the heterozygote and dominant models of the *Taq*I polymorphism was evidently related to PD risk. In addition, with a prior probability of 0.20, the *Bsm*I and *Apa*I polymorphisms were notably correlated with MCI risk (*P* < 0.2).

**TABLE 8:** False-positive report probability analysis of the noteworthy results.

SNP			Prior probability				
**Genetic modelOR (95% CI)**	***P***	**Power**	**0.25**	**0.1**	**0.01**	**0.001**	**0.0001**
**AD**							
*Fok*IAllele1.01 (0.89, 1.15)	0.881	1.000	0.725	0.888	0.989	0.999	1.000
Homozygote1.11 (0.84, 1.46)	0.455	1.000	0.577	0.804	0.978	0.998	1.000
Heterozygote0.94 (0.78, 1.13)	0.510	1.000	0.605	0.821	0.981	0.998	1.000
Dominant0.97 (0.82, 1.16)	0.739	1.000	0.689	0.869	0.987	0.999	1.000
Recessive1.11 (0.86, 1.44)	0.432	1.000	0.564	0.795	0.977	0.998	1.000
*Bsm*IAllele1.05 (0.85, 1.29)	0.642	1.000	0.658	0.853	0.985	0.998	1.000
Homozygote1.01 (0.66, 1.54)	0.963	0.999	0.743	0.897	0.990	0.999	1.000
Heterozygote1.27 (0.94, 1.73)	0.130	1.000	0.280	0.539	0.928	0.992	1.000
Dominant1.19 (0.89, 1.58)	0.229	1.000	0.407	0.673	0.958	0.996	1.000
Recessive0.88 (0.60, 1.28)	0.504	1.000	0.602	0.820	0.980	0.998	1.000
*Taq*IAllele0.87 (0.65, 1.18)	0.370	1.000	0.526	0.769	0.973	0.997	1.000
Homozygote0.67 (0.49, 0.93)	0.017	0.960	0.050*	0.135*	0.632	0.946	0.994
Heterozygote0.91 (0.63, 1.34)	0.633	0.999	0.655	0.851	0.984	0.998	1.000
Dominant0.90 (0.60, 2.49)	0.839	0.871	0.743	0.897	0.990	0.999	0.999
Recessive0.78 (0.58, 1.05)	0.101	0.998	0.233	0.477	0.910	0.990	0.999
*Apa*IAllele0.85 (0.73, 0.99)	0.037	1.000	0.099*	0.243	0.780	0.973	0.997
Homozygote0.68 (0.47, 0.96)	0.028	0.960	0.081*	0.210	0.745	0.967	0.997
Heterozygote0.88 (0.58, 1.34)	0.551	0.996	0.624	0.833	0.982	0.998	1.000
Dominant0.90 (0.70, 1.15)	0.400	1.000	0.545	0.782	0.975	0.998	1.000
Recessive0.72 (0.56, 0.92)	0.001	0.998	0.025*	0.072*	0.461	0.896	0.989
**PD**							
*Fok*IAllele0.92 (0.77, 1.08)	0.3081	1.000	0.480	0.735	0.968	0.997	1.000
Homozygote0.81 (0.56, 1.16)	0.250	0.996	0.430	0.693	0.961	0.996	1.000
Heterozygote1.09 (0.85, 1.39)	0.487	1.000	0.594	0.814	0.980	0.998	1.000
Dominant0.99 (0.82, 1.21)	0.922	1.000	0.734	0.892	0.989	0.999	1.000
Recessive0.76 (0.53, 1.09)	0.136	0.989	0.292	0.553	0.932	0.993	0.999
*Bsm*IAllele1.05 (0.96, 1.14)	0.245	1.000	0.424	0.688	0.960	0.996	1.000
Homozygote1.09 (0.91, 1.31)	0.358	1.000	0.518	0.763	0.973	0.997	1.000
Heterozygote1.09 (0.95, 1.25)	0.217	1.000	0.395	0.662	0.956	0.995	1.000
Dominant1.09 (0.95, 1.24)	0.190	1.000	0.363	0.631	0.950	0.995	0.999
Recessive1.02 (0.87, 1.19)	0.880	1.000	0.706	0.878	0.988	0.999	1.000
*Taq*IAllele1.00 (0.93, 1.09)	0.965	1.000	0.743	0.897	0.990	0.999	1.000
Homozygote0.96 (0.80, 1.14)	0.642	1.000	0.658	0.852	0.984	0.998	1.000
Heterozygote1.24 (0.99, 1.54)	0.051	1.000	0.134*	0.317	0.836	0.981	0.998
Dominant1.13 (1.01, 1.27)	0.040	1.000	0.108*	0.266	0.799	0.976	0.998
Recessive0.84 (0.66, 1.08)	0.174	1.000	0.343	0.610	0.945	0.994	0.999
*Apa*IAllele1.09 (0.80, 1.48)	0.581	1.000	0.635	0.839	0.983	0.998	1.000
Homozygote0.99 (0.59, 1.66)	0.970	0.995	0.745	0.898	0.990	0.999	1.000
Heterozygote1.13 (0.71, 1.79)	0.603	0.993	0.646	0.845	0.984	0.998	1.000
Dominant1.10 (0.68, 1.80)	0.704	0.991	0.681	0.865	0.986	0.999	1.000
Recessive0.94 (0.71, 1.26)	0.679	1.000	0.671	0.859	0.985	0.999	1.000
**MCI**							
*Fok*IAllele0.95 (0.75, 1.19)	0.655	1.000	0.663	0.855	0.985	0.998	1.000
Homozygote0.87 (0.54, 1.43)	0.583	0.986	0.640	0.842	0.983	0.998	1.000
Heterozygote1.17 (0.80, 1.72)	0.425	0.997	0.561	0.793	0.977	0.998	1.000
Dominant1.07 (0.74, 1.54)	0.780	0.995	0.702	0.876	0.987	0.999	1.000
Recessive0.79 (0.54, 1.17)	0.553	0.875	0.654	0.850	0.984	0.998	1.000
*Bsm*IAllele0.56 (0.41, 0.75)	0.000	0.776	0.000*	0.001*	0.013*	0.114*	0.563
Homozygote0.40 (0.13, 1.19)	0.100	0.344	0.464	0.722	0.966	0.997	1.000
Heterozygote0.49 (0.32, 0.75)	0.001	0.463	0.007	0.019	0.179	0.688	0.957
Dominant0.48 (0.31, 0.73)	0.000	0.424	0.004*	0.013*	0.123*	0.586	0.934
Recessive0.54 (0.33, 0.89)	0.016	0.619	0.071*	0.185*	0.715	0.962	0.996
*Taq*IAllele1.19 (0.84, 1.70)	0.339	0.998	0.505	0.754	0.971	0.997	1.000
Homozygote2.35 (0.92, 6.04)	0.076	0.369	0.382	0.650	0.953	0.995	1.000
Heterozygote0.93 (0.60, 1.44)	0.745	0.997	0.691	0.871	0.987	0.999	1.000
Dominant1.04 (0.68, 1.59)	0.856	0.999	0.720	0.885	0.988	0.999	1.000
Recessive2.41 (0.97, 6.00)	0.059	0.344	0.339	0.606	0.944	0.994	0.999
*Apa*IAllele1.37 (1.12, 1.67)	0.002	1.000	0.005*	0.016*	0.154*	0.647	0.948
Homozygote1.92 (1.24, 2.97)	0.003	0.573	0.017*	0.050*	0.369*	0.855*	0.983*
Heterozygote1.24 (0.92, 1.67)	0.157	0.999	0.320	0.585	0.939	0.994	0.999
Dominant1.37 (1.03, 1.81)	0.027	0.996	0.075*	0.195*	0.727	0.964	0.996
Recessive1.72 (1.17, 2.52)	0.005	0.781	0.020*	0.058*	0.406	0.873	0.986

*P < 0.2.

RETRACTED

## 4 Discussion

Vitamin D is an essential fat-soluble hormone that can be synthesized by skin synthesis through exposure to sunlight or dietary intake. It is involved in calcium homeostasis, cellular apoptosis, proliferation, differentiation, immunoregulation, and neuron protection (de Viragh et al., 1989; Garcion et al., 2002; Fernandes de Abreu et al., 2009). Besides, it is implicated in the brain function, exerting an important role in neuronal damage and neuroprotection (Cekic et al., 2009). Accumulative evidence has shown that vitamin D deficiency significantly attenuated the affinity of VDR to vitamin D, influenced the development, maintenance, and survival of neurons, and impaired other treatment of traumatic brain injury, resulting in neurodegeneration, neuronal aging and damage, which predicts a high risk of neurodegenerative diseases (Valdivielso and Fernandez, 2006; Vinh Quôc Luong and Thi Hoàng Nguyên, 2012). Mechanistically, vitamin D could upregulate the expression of microtubule-associated protein-2 (MAP2), growth-associated protein-43 (GAP43) and synapsin-1, induce Ca^2+^-binding protein synthesis in the cortex and hippocampus, and avoid calcium excitotoxicity, leading to clearance of brain Aβ, antioxidant and anti-inflammatory process (Taniura et al., 2006; Schlögl and Holick, 2014; Assmann et al., 2015; Landel et al., 2016). It has been reported that patients with AD, PD, and MCI have lower serum vitamin D level than age-matched control subjects, and its level was related to the severity of symptom (Sleeman et al., 2017; Larsson et al., 2018).

As a member of the nuclear steroid hormone receptor superfamily, VDR exerts a pivotal function in various biological processes (Weyts et al., 2004). VDR gene is located on the chromosome 12q13 with 2 promoter regions and 14 exons spanning approximately 75 kb (Gardiner et al., 2004; Marshall et al., 2012; Nurminen et al., 2018). It is widely expressed in the hypothalamus and in the dopaminergic neurons of substantia nigra (Eyles et al., 2005). Upon binding to the active form 1,25(OH)_2_D_3_, VDR is activated and interacts with vitamin D responsive elements in the promoters of vitamin D target genes to modulate their expression, increasing the translational efficiency (Mohri et al., 2009; Pan et al., 2009). Genetic variability in VDR could potentially affect vitamin D function and change affinity of the receptor, resulting in serious defects of receptor activation (Cai et al., 1993; Bouillon et al., 1998). Recent studies found that mice knockout VDR had muscular and locomotor impairments, but preserved the cognitive function (Burne et al., 2005). The VDR gene was prominently downregulated in the development of AD, PD, and MCI, and its expression is negatively related to the progression of these diseases (Gatto et al., 2016). It has been proposed that the expression level of VDR mRNA could be considered as a potential blood biomarker for these diseases (Scherzer et al., 2007; Wang et al., 2020).

RETRACTED

It is generally accepted that different VDR polymorphisms have potential impact on VDR expression and vitamin D levels. Studies indicated that the *Fok*I CC genotype carriers require a notably lower dose of 1,25-dihydroxyvitamin D3 than the CT genotype carriers by 50% (Colin et al., 2000). Similarly, the *Fok*I C-allele carriers possessed higher capacity for intestinal calcium absorption, leading to higher vitamin D levels (Arai et al., 1997; Uitterlinden et al., 2004). A previous study demonstrated that the *Taq*I and *Apa*I polymorphisms were not correlated with AD risk in populations with a high sun exposure in view of the higher endogenous vitamin D production, rendering the VDR activity less dependent to its amount (Łaczmański et al., 2015). Moreover, the *Taq*I polymorphism did not cause any statistically significant difference in the serum vitamin D levels nor was it related to an enhanced risk of developing AD (Oliveira et al., 2018). It has been reported that the *Taq*I TT genotype had a 1.8-fold higher likelihood of developing AD, and the potential reason may be attributed to insufficient vitamin D effects associated with the TT genotype, resulting in lower VDR affinity and VDR mRNA expression levels (Dimitrakis et al., 2022b).

A total of 30 articles covering 81 studies were included in this meta-analysis to investigate possible genetic relationships between VDR SNPs and the risk of AD, PD, and MCI. Of these studies, 10 studies were involved in AD risk, 16 studies in PD risk, and 5 studies in MCI risk, respectively. Our findings confirmed an association of *Taq*I polymorphism and AD risk among Caucasians, and a negative relationship between *Apa*I polymorphism and AD risk in the allelic, homozygous and recessive models. Except for the dominant model of *Taq*I, we did not find any remarkable correlations between other three VDR gene polymorphisms and PD risk. Subsequently, the results indicated that VDR *Bsm*I polymorphism was significantly linked with decreased MCI risk in Asian population, while the *Apa*I polymorphism was closely associated with elevated MCI risk in Caucasians and Asians. As for the MCI risk, the *Bsm*I variant might confer a protective factor in the Asian population, but the *Apa*I variant served as a hazard factor among Caucasians and Asians. In addition to possible genetic heterogeneity between different ethnicity, the result difference could be explained by difficulties in measuring serum vitamin D status and determining the actual age at onset of disease.

RETRACTED

Although VDR gene polymorphisms are a determinant of the VitD status, they act together on other genetic and environmental factors that are affected by sun exposure and diet. Genetic factors could mediate the influence of environmental factors on VDR regulation (Saccone et al., 2015). It is hypothesized that VDR gene polymorphisms takes part in the regulation of VDR activity, and the response to vitamin D supplementation varies widely between individuals (Barger-Lux et al., 1995; Arai et al., 1997). Usategui-Martín et al. demonstrated that the *Taq*I and *Fok*I variants were associated with a better response to vitamin D supplementation (Usategui-Martín et al., 2022). The *Fok*I variation exhibited a stronger impact on the response to 25(OH)D or bioavailable 25(OH)D than non-genetic factors, including body mass index, and sex (Yao et al., 2017). A randomized control study suggested that vitamin D_3_ supplementation could slow the progression of PD in patients with the *Fok*I CT and TT genotypes (Suzuki et al., 2013). The TT genotype was also found to be associated with cognitive decline in PD (Gao et al., 2020), and with PD risk (Hu et al., 2020; Agliardi et al., 2021). Importantly, understanding the genotypes of patients in advance can compensate for lower VDR availability with vitamin D supplementation to prevent the development of neurological diseases (Fan et al., 2020).

As described in previous studies, vitamin D deficiency was more common in female participants (Keeney and Butterfield, 2015; Yeşil et al., 2015). Recent studies have shown that the clinical manifestations of late-onset AD mostly occur at postmenopausal ages, and low estrogen levels are conducive to the development of the disease (Dimitrakis et al., 2022a). Due to VDR SNPs, low vitamin D levels or the poor utilization of vitamin D in postmenopausal women increased the risk of developing AD (Kinuta et al., 2000). It has been proposed that vitamin D plays a crucial role in estradiol synthesis (Enjuanes et al., 2003). Functionally, the neuroprotective effects of estrogens in neural cells against amyloid β-induced neurotoxicity are based on amyloid degradation or other molecular mechanisms (Yagyu et al., 2002; Marin et al., 2003; Quintanilla et al., 2005; Amtul et al., 2010). A cohort study indicated female patients with poor cognitive performance is associated with insufficient levels of VitD, whereas no such association was observed in male patients (Arévalo et al., 2021). The possible hypothesis is that body fat in women is greater than in men, and in this way circulating vitamin D can be stored in adipose tissue and, given its lipophilic characteristics, would be less available in plasma (Oliveira et al., 2018).

RETRACTED

There are some potential mechanisms that different VDR locus mediate the effects on diseases. VDR *Fok*I polymorphism located in exon 2 at the 5′ coding region have no linkage disequilibrium with other VDR SNPs (Gross et al., 1998). It has been found that the F-allele changes the first start codon later than the f-allele, generating a three-amino-acids shorter protein form with efficient transcription activity. However, difference in length may bring about the altered VDR function. *Bsm*I, *Apa*I (intron 8), and *Taq*I (exon 9) are located near 3′-untranslated region (3′-UTR) and then affect the expression, structure, and stability of VDR mRNA without alteration of the amino acid sequence (Ingles et al., 1997; Bretherton-Watt et al., 2001). Although the probability that these three sites directly affected VDR function is relatively low, they may be in linkage disequilibrium with genetic variability in another adjacent gene. This might influence VDR expression by altering the stability of VDR mRNA or interfering with different splicing regulatory elements (Morrison et al., 1994; Jehan et al., 1996). It has been found that the *Apa*I was in linkage disequilibrium with a poly-A repeat of the 3′-UTR and disturbed the stability of VDR mRNA, thereby affecting the cognitive function (Zmuda et al., 2000). Additionally, some underlying genes, such as CYP27A1 and CYP27B1, could affect the function of *Bsm*I, *Apa*I, and *Taq*I (Cheng et al., 2004; Uitterlinden et al., 2004). The *Apa*I genotype was found to affects the mRNA expression of target gene, including P-gp, LRP1, and RAGE, facilitating brain Aß aggregation (Arévalo et al., 2021). The Apa1 and Taq1 polymorphisms have potential interaction with interleukin-10 (IL-10) SNP, suggesting that the candidate gene may have superimposed effects with the Apa1 or Taq1 in the AD progression (Lehmann et al., 2011).

There were several inherent limitations in the present study. Firstly, the number of individual studies and sample for certain VDR SNPs were relatively low, which may restrict the statistical power and decrease the reliability of the results. Secondly, some confounding factors, including gender, serum vitamin D concentration, vitamin D supplementation, calcium intake, and time exposed to sunlight may also influence the risk of AD, PD, and MCI. The results based on unadjusted estimates for raw insufficient data might suffer from potential confounding bias. Thirdly, all the studies mainly focused on the Asian and Caucasian population, limiting the general application of the results in other populations. Lastly, different studies included in our meta-analysis used different genotyping methods for polymorphism detection. These different genotyping methods have varying sensitivity, which may potentially impact the results to a minor extent.

RETRACTED

## 5 Conclusion

In conclusion, our results indicated that VDR *Taq*I and *Apa*I polymorphisms were correlated with decreased susceptibility to AD, while no significant relationship of *Fok*I, and *Bsm*I polymorphisms with AD risk in overall analyses. Moreover, the dominant model of *Taq*I was slightly associated with PD risk. The *Bsm*I polymorphism notably decreased the MCI risk, but the *Apa*I A-allele variant significantly enhanced the MCI risk. To further elucidate the findings, studies with a better design and larger sample size are needed in the future.

## Data availability statement

The datasets presented in this study can be found in the article/Supplementary material.

## Author contributions

YD: Data curation, Investigation, Visualization, Writing – original draft. PG: Conceptualization, Data curation, Software, Visualization, Writing – original draft. QC: Methodology, Software, Validation, Writing – original draft. LH: Formal analysis, Investigation, Visualization, Writing – original draft. LL: Data curation, Software, Writing – original draft. MY: Investigation, Methodology, Software, Writing – original draft. MT: Formal analysis, Visualization, Writing – review & editing. JM: Formal analysis, Visualization, Writing – review & editing. XS: Conceptualization, Supervision, Writing – original draft. LF: Conceptualization, Project administration, Supervision, Writing – review & editing.

## Supplementary material

Supplementary Figure 1 Forest plots for the association between VDR *Fok*I polymorphism and AD risk in five models. **(A)** Allele model; **(B)** dominant model; **(C)** heterozygote model; **(D)** homozygote model; **(E)** recessive model.

Supplementary Figure 2 Forest plots for the association between VDR *Bsm*I polymorphism and AD risk in five models. **(A)** Allele model; **(B)** homozygote model; **(C)** heterozygote model; **(D)** dominant model; **(E)** recessive model.

Supplementary Figure 3 Forest plots for the association between VDR *Taq*I polymorphism and AD risk in five models. **(A)** Allele model; **(B)** homozygote model; **(C)** heterozygote model; **(D)** dominant model; **(E)** recessive model.

RETRACTED

Supplementary Figure 4 Forest plots for the association between VDR *Fok*I polymorphism and PD risk in five models. **(A)** Allele model; **(B)** homozygote model; **(C)** heterozygote model; **(D)** dominant model; **(E)** recessive model.

Supplementary Figure 5 Forest plots for the association between VDR *Apa*I polymorphism and PD risk in five models. **(A)** Allele model; **(B)** homozygote model; **(C)** heterozygote model; **(D)** dominant model; **(E)** recessive model.

Supplementary Figure 6 Forest plots for the association between VDR *Fok*I polymorphism and MCI risk in five models. **(A)** Allele model; **(B)** homozygote model; **(C)** heterozygote model; **(D)** dominant model; **(E)** recessive model.

Supplementary Figure 7 Forest plots for the association between VDR *Bsm*I polymorphism and MCI risk in five models. **(A)** Allele model; **(B)** homozygote model; **(C)** heterozygote model; **(D)** dominant model; **(E)** recessive model.

Supplementary Figure 8 Forest plots for the association between VDR *Apa*I polymorphism and MCI risk in five models. **(A)** Allele model; **(B)** homozygote model; **(C)** heterozygote model; **(D)** dominant model; **(E)** recessive model.

Supplementary Figure 9 Sensitivity analysis for VDR gene polymorphism and AD risk in dominant model. **(A)** *Fok*I polymorphism; **(B)** *Bsm*I polymorphism; **(C)** *Taq*I polymorphism; **(D)** *Apa*I polymorphism.

Supplementary Figure 10 Sensitivity analysis for VDR gene polymorphism and MCI risk in dominant model. **(A)** *Fok*I polymorphism; **(B)** *Bsm*I polymorphism; **(C)** *Taq*I polymorphism; **(D)** *Apa*I polymorphism.

Supplementary Figure 11 Begg’s funnel plot for detecting the publication bias in the dominant model of VDR SNPs. **(A)** *Fok*I polymorphism and AD risk; **(B)** *Bsm*I polymorphism and AD risk; **(C)** *Taq*I polymorphism and AD risk; **(D)** *Apa*I polymorphism and AD risk; **(E)** *Fok*I polymorphism and PD risk; **(F)** *Bsm*I polymorphism and PD risk; **(G)** *Taq*I polymorphism and PD risk; **(H)** *Apa*I polymorphism and PD risk; **(I)** *Fok*I polymorphism and MCI risk; **(J)** *Bsm*I polymorphism and MCI risk; **(K)** *Taq*I polymorphism and MCI risk; **(L)** *Apa*I polymorphism and MCI risk.

Supplementary Table 1 Newcastle-Ottawa Scale for VDR gen polymorphisms in the AD, PD, and MCI.
